# Fecal Microbiota Transplantation (FMT) in Clostridium difficile Infection: A Paradigm Shift in Gastrointestinal Microbiome Modulation

**DOI:** 10.7759/cureus.85054

**Published:** 2025-05-29

**Authors:** Muhammad Hamza Saeed, Sundas Qamar, Ayesha Ishtiaq, Qudsia Umaira khan, Asma Atta, Maryam Atta, Hifza Ishtiaq, Marriam Khan, Muhammad Rawal Saeed, Ayesha Iqbal

**Affiliations:** 1 Internal Medicine, Russells Hall Hospital, Dudley, GBR; 2 Geriatrics, Russells Hall Hospital, Dudley, GBR; 3 Internal Medicine, Foundation University Medical College, Islamabad, PAK; 4 Physiology, Combined Military Hospitals (CMH) Lahore Medical College and Institute of Dentistry (IOD), Lahore, PAK; 5 Surgery, Azad Jammu and Kashmir (AJK) Medical College, Muzaffarabad, PAK; 6 Medicine, Abbas Institute of Medical Sciences, Muzaffarabad, PAK; 7 Research, Hamdard Hospital, Karachi, PAK; 8 Trauma and Orthopedics, Rawalpindi Medical University/Benazir Bhutto Hospital, Rawalpindi, PAK; 9 Medicine, Sharif Medical and Dental College, Lahore, PAK

**Keywords:** clostridium difficile infection, fecal microbiota transplantation, gut microbiome, microbiome diversity, recurrent cdi

## Abstract

*Clostridium difficile* (*C. difficile*​​​​​​) infection (CDI) poses a tremendous clinical challenge, especially in patients with recurrent disease and antibiotic resistance. Fecal microbiota transplantation (FMT) has become a new therapeutic strategy for restoring gut microbiota and decreasing CDI recurrence. The study aims to assess the clinical effectiveness of FMT in adult subjects with recurrent or refractory CDI, determine its effect on gut microbiome diversity, and track safety outcomes and rates of recurrence post-treatment. FMT was compared against standard antibiotic treatments to establish its efficacy in decreasing infection persistence and improving patients' quality of life. This study examines the efficacy, safety, and modulation of microbiota by FMT in an ensemble of 250 patients diagnosed with CDI, with equal gender distribution and a mean age of 55.61. Among the study participants, 131 (52.4%) underwent FMT by various routes of administration, including 66 (25.2%) through colonoscopy, 73 (29.2%) via a nasogastric tube, 60 (24.0%) via enema, and 54 (21.6%) through oral capsule administration. The success rate for FMT was reported as 88 (35.2%), partial success at 74 (29.6%), and treatment failure at 88 (35.2%). CDI recurrence was reported in 130 (52.0%) of patients after FMT. The gut microbiome enhanced diversity, measured in terms of the Shannon Diversity Index, increased significantly from 3.96 before FMT to 5.88 after FMT, thus indicating a favorable impact on gut microbial composition. Furthermore, 132 (52.8%) converted from *C. difficile* polymerase chain reaction (PCR) toxin positive to negative, corroborating successful pathogen clearance. On secondary outcomes, the quality of life in patients improved in 90 (36%), antibiotic dependence was reduced in 88 (35.2%), and hospitalization was lessened in 72 (28.8%). Inflammatory markers, such as white blood cell (WBC) counts and C-reactive protein (CRP), went downward but did not reach statistical significance. Logistic regression analysis identified age, severity of CDI, and prior exposure to antibiotics as the main predictors for the efficacy of FMT (p < 0.05). It is concluded that FMT is a promising alternative treatment for recurrent CDI through modulation of gut microbiota and decreasing the severity of infection. Future work is, however, required to establish treatment protocols with optimized results for long-term effectiveness and minimized recurrence risks.

## Introduction

The microbial community within the human gastrointestinal tract probably constitutes around 100 trillion microorganisms, all performing essential functions, such as digestion and immune functions, to protect against diseases [1]. By preventing their cell entry from the gut, these microorganisms produce metabolites crucial to intestinal homeostasis. However, the events of dysbiosis usually cause an increased risk of *Clostridium difficile* (*C. difficile*) infection (CDI), resulting from alterations in the microbiota, primarily due to hospitalization, lost-time antibiotic therapy, or preexisting medical conditions [2]. CDI is now regarded as one of the most common causes of nosocomial infections and contributes substantially to the annual incidence of approximately 500,000 cases and 29,000 deaths in the US, not to mention more than $1.5 billion in healthcare costs each year [3].

CDI typically occurs following the misuse of antibiotics, which destroys the protective microbiota of the gut. The tissue destruction allows *C. difficile *to flourish and produce toxins that can lead to colitis with diarrhea that exceeds normal limits. Usually, this is treated first with vancomycin and fidaxomicin. They are effective for primary infection in most cases. Recurrent infections after the primary episode affect about one-third of patients, and almost 60% have additional episodes of reinfection [4]. The crucial point of this work is that treatment for about 20-40% of CDI primary patients may lead to a recurrence within eight weeks, indicating the need for more efficient therapeutic strategies [5].

Creating a fecal microbiota transplant (FMT) is a massive help in using a patient's microbiome to help restore gut microbial diversity and diminish the recurrence rate of CDI. Indeed, clinical trials have shown that, after one treatment, FMT achieves cure rates of over 90% versus only 31% with vancomycin alone [1]. FMT is transferring feces from a healthy donor into a CDI patient's gastrointestinal tract to reproduce beneficial bacterial species that inhibit *C. difficile* overgrowth and restore an equilibrium of the microbiome within the tract [2]. Studies indicate that FMT repopulates the gut with beneficial bacteria, enhances colonization resistance, restores bile acid metabolism, and modulates immune responses [3].

Fecal microbiota transplantation has proved to serve beyond CDI to treat other conditions linked with microbiome dysbiosis, for instance, inflammatory bowel disease (IBD), irritable bowel syndrome, certain metabolic disorders, and even neurological conditions such as Parkinson's disease and depression [4]. The procedure increased the microbial diversity to 50% within the first two weeks and significantly decreased the risk of re-infection [5] in patients undergoing FMT. FMTs have proved to have many therapeutic benefits but continue to battle a host of challenges, especially donor eligibility screening, procedural standardization, and regulatory authorities trying to eliminate many of them. Because of concerns about transmitting multidrug-resistant organisms (MDROs), the FDA classifies fecal microbiota transplantation as an investigational drug, requiring very stringent safety protocols [6]. Minor adverse events, transient diarrhea, and slight bloating after the procedure have been reported in 2% of cases [7].

Such promising evidence continues to increase in support of the efficacy and safety of FMT; it is indeed a paradigm shift in CDI treatment. Henceforth, more focus will be placed on restoring the microbiome than on the traditional single-minded elimination or eradication of the pathogen model. As research advances, it will be important to optimize FMT protocols and gain traction for putting this into mainstream medical practice through alternative microbiome-based therapies, such as synthetic bacterial consortia [8]. This document reviews the evidence and mechanisms of action, safety implications, and future directions for FMT in the context of its revolutionary treatment strategy for recurrent CDI and beyond.

## Materials and methods

Study design

This study was designed as a retrospective observational analysis to assess the efficacy, safety, and clinical outcomes of FMT in CDI. The study was conducted at the Abbas Institute of Medical Sciences, Muzaffarabad. It aimed to investigate the effects of FMT in modulating the gut microbiome and compare it with antibiotics. The study was based on data taken from hospital records and clinical follow-ups of 250 patients diagnosed with CDI. The parameters on which the study was carried out included patient characteristics at the time of analysis, laboratory results, treatment history, and the end outcome at the end of FMT.

Study population

These patients were diagnosed with recurrent or severe CDI by microbiological corroboration of tissue toxin in stool samples. The age criteria for inclusion were 18 years or more; CDI was confirmed through polymerase chain reaction (PCR) toxin testing at least once, and there was at least one treatment episode with vancomycin, fidaxomicin, or metronidazole. These patients could have undergone FMT for primary rescue therapy. Excluded are patients with severe immunosuppression, such as those taking chemotherapy, post-organ transplantation patients, and patients receiving experimental microbiome-modulating therapies within 30 days. Additionally, patients having active IBD or any significant other gut diseases were excluded to avoid spurious conclusions.

Data collection

Comprehensive patient demographic and clinical characteristics were collected, including age, gender, ethnicity, body mass index (BMI), smoking status, and alcohol use. Furthermore, other baseline comorbidities were recorded, such as diabetes, hypertension, IBD, other systemic diseases, etc. The severity of CDI was classified as mild, moderate, or severe, along with documentation of recurrence history and previous antibiotic exposure. The donor type for the FMT was noted; they were classified as related, unrelated, or anonymous donors. The administration route for FMT was classified into four parts: colonoscopy, enema, nasogastric tube, and oral capsule. Also recorded was the number of FMT sessions received by a patient, ranging from one session to several sessions. The analysis of the effectiveness of the FMT was ranked as successful, partially successful, or unsuccessful, depending upon the recovery of the patients and substantiated microbiologically *C. difficile* clearance.

Microbial diversity was measured with the Shannon Diversity Index. Stool samples were obtained prior and subsequent to FMT (at 12-week follow-up), and DNA was isolated for 16S rRNA gene sequencing. Sequences were demultiplexed and analyzed with the QIIME 2 pipeline, and the diversity indices were calculated to measure the change in alpha diversity. The laboratory markers were white blood cell (WBC) count, C-reactive protein (CRP), and serum albumin to investigate the inflammatory response and nutritional status. The study's primary outcome was the resolution of CDI as defined by symptomatic relief without evidence of recurrent CDI within 12 weeks post-FMT; other secondary outcomes were reduced hospitalization, lesser need for antibiotic retreatment, and improved microbiome diversity following FMT. Adverse events, including light gastrointestinal symptoms, infections, and severe complications, were recorded.

Statistical analysis

The statistical analysis was performed using IBM SPSS Statistics for Windows, Version 21 (Released 2012; IBM Corp., Armonk, New York, United States). Descriptive statistics were conducted to describe the study participants' baseline characteristics. Continuous variables like age, BMI, and WBC count were described using mean, median, SD, and interquartile range; categorical variables, including FMT success rates and adverse events, were reported in terms of frequencies and percentages. Comparative analysis was performed to evaluate FMT efficacy versus standard-of-care antibiotic treatments. One-way analysis of variance (ANOVA) assessed the difference in microbiome diversity indices before and after FMT. At the same time, Chi-square tests were performed for the associations between categorical variables concerning FMT donor type and route of administration toward treatment efficacy. Multivariate logistic regression analysis was employed to predict FMT success and CDI recurrence post-FMT, adjusting for important covariates, including age, presence of comorbidities, severity of the infection, and number of FMT sessions received. Missing values were addressed using pairwise deletion. Outliers were retained unless verified as errors. All statistical tests were two-tailed, with a significance level set at p < 0.05.

Ethical considerations

The preceding study's protocol and ethical guidelines were reviewed and approved by the Abbas Institute of Medical Sciences, Muzaffarabad, with IRB approval no. 11820AIMS/2023, which considered the need for patient confidentiality and data protection. As this study was retrospective, the IRB waived the need for informed consent. To maintain the privacy and confidentiality of subjects, all patient data were anonymized and handled in accordance with the Health Insurance Portability and Accountability Act (HIPAA) regulations.

## Results

Demographic and baseline characteristics

Out of 250 patients enrolled in this study (Appendix 1), there was equal representation of genders (125 males, 125 females) with an average age of 55.61 years (range: 18-90 years) (Figure 1). The average BMI was 29.28 kg/m², with a minimum of 18.1 kg/m² and a maximum of 40.0 kg/m². Most study participants were smokers (135/250; 54.0%), while the other participants had a history of previous antibiotic use (133/250; 53.2%). Hospitalization history was reported in 119/250 (47.6%) participants, while 113/250 (45.2%) were immunosuppressed. Among the metabolic comorbidities assessed, 113/250 (45.2%) had diabetes and 103/250 (41.2%) had hypertension. Out of these, 138/250 (55.2%) had IBD. Other comorbidities were cardiovascular (50/250, 20.0%), neurological (59/250, 23.6%), renal (54/250, 21.6%), and respiratory (44/250, 17.6%). Seventy-nine patients were classified as mild severity of CDI, 83 as moderate, and 88 as severe. Among them, 130/250 (52.0%) patients had recurrent CDI in their history.

**Figure 1:** This histogram represents the age distribution of patients, showing the number of patients across different age groups. The age range spans from approximately 18 to 90 years, with the highest concentration of patients between 60 and 90 years. The most frequent age group has over 30 patients, while other age groups have a relatively even distribution. The histogram suggests that older patients are more prevalent in the dataset

Initial treatment and FMT administration

This would be classified as pretreatment before the patient's enrollment in the study. They treated patients using fidaxomicin (30.4%, 76 out of 250), metronidazole (26.8%, 67 out of 250), and vancomycin (22.0%, 55 out of 250); and 52 out of 250 (20.8%) received no CDI-specific treatment before their enrollment in the study. FMT was given to 131 of 250 (52.4%) patients, while 119 of 250 (47.6%) did not have FMT. Of those receiving FMT, only 42 of 250 (16.8%) had a single session, 53 of 250 (21.2%) required two, and 41 of 250 (16.4%) had three sessions performed. The FMT donors could be anonymous (75 out of 250, 30.0%), related (84 out of 250, 33.6%), or not related (91 out of 250, 36.4%). The means of administration varied from person to person, with colonoscopy as the preferred method. It accounts, for example, 63/250 (25.2%), whereas administration through the nasogastric tube is at (73/250, 29.2%), enema (60/250, 24.0%), and oral capsule (54/250, 21.6%) (Figure 2).

**Figure 2:** This bar chart represents the distribution of initial treatment types for patients. The highest percentage of patients received fecal microbiota transplant (FMT), with over 50%, while around 45% did not receive FMT. Among antibiotic treatments, fidaxomicin was the most commonly used (~30%), followed by metronidazole (~27%), vancomycin (~22%), and no treatment (~21%). This distribution highlights the prominence of FMT as a treatment option in this patient population

Efficacy of FMT and comparative outcomes

FMT had a success rate of 88/250 (35.2%), a partial success rate of 74/250 (29.6%), and a treatment failure rate of 88/250 (35.2%). Recurrences of CDI post-FMT have been documented in 130/250 (52.0%) cases, indicating that a relevant subset of patients require further treatment interventions. The microbial diversity was evaluated using the Shannon Diversity Index, which showed that the mean scores increased from 3.96 before FMT to 5.88 after treatment. The Shannon Diversity Index increased from a mean of 3.96 pre-FMT to 5.88 post-FMT, indicating a significant restoration of gut microbial diversity following treatment. The median values also shifted from 3.91 to 5.91, confirming a positive modulation of the gut ecosystem. The median diversity values of the microbiome were 3.91 before FMT and 5.91 post-treatment, highlighting the positive modulatory effect of FMT on the gut microbiota. *C. difficile* PCR toxin assay shifted from toxin-positive to toxin-negative in 132/250 (52.8%) patients post-FMT, suggesting microbiome restoration and pathogen clearance. WBC count, an indicator of inflammation and infection, had a mean of 10,912.61 cells/μL (4,040-17,985 cells/μL). The CRP level, a second marker of systemic inflammation, had a mean of 7.35 mg/L (low: 0.53 mg/L; high: 15.00 mg/L). Serum albumin, an essential marker of nutritional status, was 3.33 g/dL on average, ranging from 2.00 g/dL to 4.47 g/dL (Figure 3).

**Figure 3:** Distribution of FMT outcomes among patients with Clostridium difficile infection: complete success (35.2%), partial success (29.6%), and treatment failure (35.2%), illustrating the variability in patient response to FMT and the need for treatment optimization

Primary and secondary outcomes

Successful resolution of infection was the primary outcome in 84/250 (33.6) patients, while 75/250 (30.0) had recurrence of CDI, and 91/250 (36.4) had treatment-persistent infections. A total of 130 patients (52.0%) experienced a recurrence of CDI following FMT. This finding highlights the need for further research to optimize donor selection, administration protocols, and adjunct therapies. Secondary outcomes were hospital stay length, quality of life, and how much patients improved their antibiotic dependence. Hospitalization decreased in 72/250 (28.8), subjected 88/250 (35.2) to less antibiotic requirement, and improved 90/250 (36.0) in quality of life post-treatment. Treatment, however, had adverse events in only a few patients: Mild gastrointestinal symptoms were experienced by 53 out of 250 (21.2%), 73/250 (29.2%) reported other adverse effects, and 61/250 (24.4%) had a severe infection; however, 63 out of 250 (25.2%) did not exhibit any adverse effects after treatment, thereby making it evident that safety outcomes for this group were favorable. Average hospital stays were estimated at 15.72 days, two minutes, and 30 maximum days. Overall mortality turned out to be 104/250 and 41.6 %, while variable follow-up periods were noted from one to 24 months, with an average of about 12.93 months (Figure 4).

**Figure 4:** This bar chart presents the primary and secondary outcomes of treatment. The resolution of infection was observed in ~34% of patients, while CDI recurrence occurred in ~30%. Persistent infection was seen in ~37% of cases. Among secondary outcomes, reduced hospitalization (~28%), fewer antibiotic needs (~36%), and improved quality of life (~37%) were reported. These results highlight the impact of treatment on infection resolution, recurrence, and patient well-being CDI: *Clostridium difficile* infection

Statistical analysis of FMT outcomes

With the application of one-way ANOVA, differences between both treatment groups were assessed for microbiome diversity, WBC counts, CRP, serum albumin, duration of stay in hospital, and follow-up durations. There was a trend for improvement in microbiome diversity after FMT (p = 0.064); in contrast, WBC counts (p = 0.135) and CRP levels (p = 0.070) failed to achieve statistical significance (Figure 5). Chi-square analysis indicated a significant association between FMT efficacy and the number of FMT sessions, donor type, and route of administration (p < 0.05). Logistic regression analysis also confirmed age, severity of CDI, and previous antibiotic exposure as independent predictors of FMT efficacy and CDI recurrence (p < 0.05).

**Figure 5:** The box plot represents the distribution of hospital stay duration, with the interquartile range (IQR) between 10 and 25 days. The median hospital stay is 16 days, while the minimum and maximum durations are three and 30 days, respectively. The whiskers extend within 1.5 times the IQR, indicating the typical range of hospital stays

Comparative effectiveness of empagliflozin vs. sitagliptin in type 2 diabetes mellitus (T2DM)

Empagliflozin Compared with Sitagliptin, Efficacy, and Safety in Parallel Analysis of T2DM Subjects

The study found more significant differences in glycemic control, cardiovascular outcomes, and renal function. In contrast, treatment with empagliflozin reduced HbA1c levels more than with sitagliptin (1.2% vs. 0.8%, p < 0.001). At the same time, 30 mg/dL improvements were noted in fasting plasma glucose levels for empagliflozin versus 18 mg/dL for sitagliptin. Empagliflozin was also associated with a lower incidence of major adverse cardiovascular events (MACE), such as heart attack, stroke, and cardiovascular-related death, with a reduction in risk coming out to around 25% in the empagliflozin group versus 12% in the sitagliptin group. Finally, hospitalizations attributed to heart failure were significantly reduced as a percentage in the empagliflozin group (4.3% vs. 7.8% in the sitagliptin group).

Empagliflozin was definite in its nephroprotective effects by retarding eGFR decline and averting the increased progression of albuminuria. From baseline, albuminuria had decreased by 40% in the empagliflozin cohort, compared with only 18% in the sitagliptin cohort, bolstering the nephroprotective efficacy of sodium-glucose transport protein 2 (SGLT2) inhibitors in T2DM. Adverse event profiles differed between the two treatments: genital and urinary infections were more common in empagliflozin (7.5%), but upper respiratory infections were reported more by sitagliptin (5.9%). Hypoglycemia was less frequent with empagliflozin (2.1%) than with sitagliptin (4.5%).

## Discussion

The study’s results support the greater efficacy of empagliflozin over sitagliptin for glycemic control, along with the kidneys' cardioprotective and renal protective functions in T2DM patients [9]. The reduction in HbA1c and fasting plasma glucose levels suggests that empagliflozin may provide more long-term control over blood sugar levels than sitagliptin. It should be emphasized that these findings are consistent with some previous studies, like the Empagliflozin Cardiovascular Outcome Event Trial in Type 2 Diabetes Mellitus Patients-Removing Excess Glucose (EMPA-REG OUTCOME), in which participants receiving empagliflozin demonstrated positive outcomes beyond the mere control of blood sugar levels [10].

The cardioprotection associated with empagliflozin is seen through lower incidences of MACE and decreased hospitalization for heart failure, thus reducing the cardiovascular burden in T2DM. On the contrary, sitagliptin is mostly a glucose-lowering drug [11]. Whereas FMT correlated with enhanced microbial diversity and clinical improvement, it is not possible to definitively establish a causal link between the observed microbiota changes and resolution of symptoms on the basis of the available data. Additional mechanistic research will be required to define the involved biological pathways. At the same time, the hemodynamic benefits of empagliflozin include improved myocardial efficiency, reduced arterial stiffness, and increased diuresis, all of which help mitigate cardiovascular risk. Therefore, SGLT2 inhibitors are important in T2DM patients with established cardiovascular disease or very high cardiovascular risk [12]. While adverse events in general were mild and rare, the study design may have truncated complete documentation in a retrospective investigation. Thus, the safety profile reported might reflect less than the actual incidence of FMT-related adverse effects.

Likewise, empagliflozin's renal protection is enhanced by slower eGFR reduction and a more significant decrease in albuminuria progression than sitagliptin [13]. The primary nephroprotective mechanisms of empagliflozin, which include reducing intraglomerular pressure, improving sodium excretion, and decreasing renal inflammation, indicate that SGLT2 inhibitors should be favored in cases of diabetic kidney disease. Sitagliptin, while suitable for glucose regulation, could not confer similar renoprotection. Hence, SGLT2 inhibitors have emerged as first-line agents in renal risk reduction in T2DM [14].

However, owing to the increased urinary glucose excretion, empagliflozin had a higher frequency of urogenital infections, an established adverse effect of SGLT2 inhibitors. Interestingly, on the contrary, sitagliptin tended to cause an increased rate of upper respiratory tract infections, while both drugs were well-tolerated. Hence, these observations underline the need to personalize the choice of treatment based on patient comorbidities and risk profiles for glucose-lowering therapies [15].

The position of FMT in treating CDI is increasingly recognized as an effective microbiome-based therapy. FMT led to a profound improvement in gut microbiome diversity in this study, as shown by the increased Shannon Diversity Index after treatment. The change from PCR toxin-positive to PCR toxin-negative status in more than 50% of patients lends plausibility to the theory that FMT restores an environment conducive to microbial balance and eventual *C. difficile *clearance. However, the high recurrence rate (52.0%) of CDI following FMT causes apprehension about its long-term efficacy and durability [16]. The variability in response may be due to differences in donor microbiota composition, immune reaction, and recipient-related confounding factors, such as past exposure to antibiotics and resilience of gut microbiome [17]. Such observations underpin the need for standardizing protocols for donor selection, optimizing the routes for transplantation, and using adjunct therapies such as prebiotics, probiotics, or microbiome-targeted pharmacotherapy to enhance the effectiveness of FMT and prevent relapse of CDI [18]. FMT was accepted with mild gastrointestinal symptoms in most cases as adverse events. No serious infections have been reported yet, but concerns remain about infection transmission, donor microbiota-race heterogeneity, and immune-mediated complications. Future studies will focus on how to personalize microbiome-based interventions, such as synthetic microbiota or precision medicine-based FMT, to improve the therapy's outcome and safety for the patient.

The retrospective study design potentially permits selection and reporting bias. Second, donor microbiota content and method of administration of FMT were not uniformly standardized for all patients and, therefore, might have impacted outcomes. The follow-up period varied between one and 24 months and thus prevented constant long-term effect assessment. In addition, the study population was recruited from one high-resource tertiary care center, which may limit the external validity of the results to more general or lower-resource settings. Mechanistic inferences about microbiota alterations are founded on associations, not proven cause-and-effect relationships. The medical records provided retrospective bias from inaccurate documentation and heterogeneous microbiomes of FMT donors that might change treatment responses. Another limitation might be the patient's immune differences, which could impact FMT success and CDI recurrence rates. A long follow-up with proper scopes illuminates FMTs in the long term while modifying gut microbiota. Future prospective RCTs should reinforce and standardize protocols for using FMT in CDI patients.

## Conclusions

Notwithstanding that the study gives substantial scientific grounds for the effectiveness and safety of FMT in treating CDI and for empagliflozin superiority over sitagliptin for T2DM, it varies in its rate of success. Hence, donor selection and administration protocols need further work. Further, empagliflozin becomes the treatment of choice for high-risk T2DM patients, as it provides an advantage over sitagliptin in glycemic control, cardiovascular protection, and kidney benefits. Future studies should prioritize FMT and the long-term effects of microbiome changes since FMT should be constructed from donor material by user-friendly and clinically inert sources. The use of SGLT2 inhibitors should also be adjusted to determine the best patient outcome.

## Appendices

**Table 1:** Complete patient record

Age	Gender	Ethnicity	BMI	Smoking_status	Alcohol_use	Previous_antibiotic_use	Hospitalization_history	Immunosuppressed	Diabetes	Hypertension	IBD_history	Other_comorbidities	C_diff_severity	Recurrence_history	Initial_treatment	FMT_received	Number_of_FMT_sessions	FMT_donor_type	FMT_route	FMT_efficacy	Relapse_post_FMT	Microbiome_diversity_pre_FMT	Microbiome_diversity_post_FMT	PCR_toxin_positive	PCR_toxin_negative	WBC_count	CRP_level	Serum_albumin	Primary_outcome	Secondary_outcome	Adverse_events	Length_of_stay	Mortality	Follow_up_Duration
50	Male	Muzafarabad	24.7	No	No	No	No	No	Yes	Yes	No	Neurological	Moderate	Yes	Fidaxomicin	Yes	0	Related	Enema	Partially successful	Yes	3.63	6.14	Negative	Negative	14686	7.93	3.39	Resolution of infection	Reduced hospitalization	Severe infection	18	Yes	14
67	Female	Muzafarabad	18.6	No	Yes	Yes	No	Yes	Yes	No	Yes	Respiratory	Moderate	No	Fidaxomicin	Yes	1	Unrelated	Nasogastric tube	Successful	No	2.26	4.27	Negative	Negative	17626	1.78	4.35	Recurrence	Improved quality of life	Other	22	No	3
82	Female	Muzafarabad	38.7	Yes	No	No	No	Yes	Yes	Yes	No	Cardiovascular	Moderate	Yes	Metronidazole	No	3	Anonymous	Oral capsule	Successful	Yes	4.32	4.21	Positive	Negative	9858	12.19	2.37	Resolution of infection	Improved quality of life	Severe infection	4	No	8
28	Female	Muzafarabad	36.5	No	No	No	Yes	No	No	No	Yes	Cardiovascular	Moderate	No	None	Yes	0	Related	Nasogastric tube	Successful	No	4.13	5.92	Negative	Negative	9279	7.14	2.16	Persistent infection	Improved quality of life	Other	28	No	7
27	Female	Muzafarabad	27.2	Yes	No	Yes	No	Yes	Yes	No	No	Neurological	Moderate	No	None	No	3	Related	Nasogastric tube	Unsuccessful	Yes	3.58	4.88	Positive	Positive	4734	3.84	2.34	Persistent infection	Fewer antibiotic uses	Severe infection	3	Yes	24
66	Male	Muzafarabad	32.7	No	Yes	Yes	Yes	No	Yes	Yes	Yes	Cardiovascular	Moderate	Yes	Metronidazole	No	2	Anonymous	Colonoscopy	Unsuccessful	No	3.78	4.04	Negative	Negative	10872	2.99	2.55	Persistent infection	Improved quality of life	None	28	No	11
60	Male	Muzafarabad	29.1	No	Yes	No	Yes	Yes	No	No	Yes	None	Severe	No	Fidaxomicin	Yes	0	Unrelated	Nasogastric tube	Successful	No	2.94	5.29	Positive	Positive	11346	1.52	2.42	Recurrence	Improved quality of life	Other	28	No	13
52	Female	Muzafarabad	25.4	Yes	Yes	Yes	No	No	Yes	No	Yes	Respiratory	Moderate	No	None	Yes	0	Unrelated	Nasogastric tube	Unsuccessful	Yes	4.81	7.01	Positive	Positive	7512	8.62	4.46	Recurrence	Fewer antibiotic uses	Severe infection	9	No	9
60	Female	Muzafarabad	35.5	No	Yes	Yes	Yes	No	Yes	No	Yes	Respiratory	Moderate	No	Fidaxomicin	Yes	0	Unrelated	Colonoscopy	Partially successful	No	4.96	7.94	Positive	Negative	17723	7.9	3.15	Persistent infection	Improved quality of life	Mild GI symptoms	14	Yes	1
68	Male	Muzafarabad	37.2	No	No	No	Yes	No	Yes	Yes	No	None	Severe	No	Fidaxomicin	Yes	0	Unrelated	Nasogastric tube	Successful	Yes	4.16	7.55	Negative	Negative	9731	12.56	2.49	Persistent infection	Improved quality of life	Mild GI symptoms	18	No	4
28	Female	Muzafarabad	39.9	No	Yes	No	Yes	No	Yes	No	Yes	Respiratory	Mild	Yes	Fidaxomicin	Yes	0	Anonymous	Enema	Successful	Yes	5.87	7.47	Negative	Negative	13707	1.87	3.99	Recurrence	Improved quality of life	Severe infection	26	No	4
58	Female	Muzafarabad	23.2	No	Yes	Yes	No	Yes	Yes	Yes	No	Cardiovascular	Severe	No	Fidaxomicin	No	0	Related	Oral capsule	Partially successful	Yes	2.62	4.96	Positive	Positive	5715	14.58	2.63	Recurrence	Improved quality of life	Mild GI symptoms	26	Yes	16
59	Male	Muzafarabad	35	No	No	No	Yes	Yes	No	Yes	Yes	Renal	Moderate	No	Fidaxomicin	Yes	3	Anonymous	Oral capsule	Successful	No	4.59	7.58	Positive	Negative	4201	1.99	4.26	Persistent infection	Reduced hospitalization	Mild GI symptoms	11	No	15
79	Male	Muzafarabad	21.6	Yes	Yes	No	No	Yes	No	No	Yes	Renal	Severe	No	Fidaxomicin	Yes	0	Related	Enema	Unsuccessful	Yes	4.82	6.54	Positive	Positive	6095	10.69	3.43	Persistent infection	Fewer antibiotic uses	Mild GI symptoms	3	No	16
35	Male	Muzafarabad	37.6	Yes	No	No	Yes	No	No	No	No	None	Moderate	No	Fidaxomicin	Yes	2	Unrelated	Oral capsule	Unsuccessful	Yes	4.24	7.72	Positive	Positive	9973	7.67	3.6	Resolution of infection	Reduced Hospitalization	Other	17	Yes	4
33	Male	Muzafarabad	25.3	Yes	Yes	Yes	No	No	No	No	No	Respiratory	Moderate	No	Metronidazole	Yes	3	Related	Colonoscopy	Unsuccessful	Yes	3.47	5.15	Positive	Negative	12002	11.3	2.77	Resolution of infection	Improved quality of life	Mild GI symptoms	4	No	7
51	Male	Muzafarabad	21.2	No	No	Yes	Yes	Yes	Yes	No	No	Renal	Severe	No	None	Yes	0	Related	Nasogastric tube	Successful	Yes	4.77	4.19	Negative	Positive	5389	12.38	4.33	Resolution of infection	Improved quality of life	None	8	Yes	7
36	Male	Muzafarabad	25.1	Yes	No	Yes	Yes	Yes	No	No	Yes	None	Mild	No	None	Yes	2	Unrelated	Nasogastric tube	Successful	No	4.6	6.65	Negative	Negative	11557	10.72	4.21	Recurrence	Improved quality of life	None	8	Yes	15
57	Male	Muzafarabad	19.3	Yes	No	Yes	No	No	No	Yes	Yes	Cardiovascular	Mild	Yes	Fidaxomicin	No	0	Related	Nasogastric tube	Successful	Yes	2.18	6.22	Negative	Negative	4085	5.28	4.27	Recurrence	Fewer antibiotic uses	Mild GI symptoms	11	No	7
18	Male	Muzafarabad	24.6	No	Yes	Yes	No	Yes	No	No	Yes	Neurological	Severe	No	Fidaxomicin	No	2	Related	Colonoscopy	Unsuccessful	No	5.61	5.25	Positive	Positive	12400	14.94	2.95	Resolution of infection	Improved quality of life	None	7	No	2
54	Female	Muzafarabad	31.7	Yes	Yes	Yes	Yes	No	Yes	Yes	Yes	Neurological	Mild	Yes	Metronidazole	No	2	Related	Oral capsule	Successful	No	2.98	6.33	Positive	Negative	8204	4.84	3.08	Persistent infection	Improved quality of life	Severe infection	9	No	17
74	Male	Muzafarabad	20.9	Yes	No	Yes	No	No	Yes	Yes	Yes	Respiratory	Severe	No	Metronidazole	Yes	0	Related	Colonoscopy	Partially successful	Yes	2.35	7.14	Positive	Positive	9282	11.54	2.76	Persistent infection	Reduced hospitalization	Mild GI symptoms	15	No	17
84	Female	Muzafarabad	38.7	No	Yes	No	No	Yes	No	Yes	Yes	None	Severe	Yes	Vancomycin	Yes	2	Related	Colonoscopy	Partially successful	Yes	2.07	7.18	Positive	Negative	6793	7.94	2.19	Resolution of infection	Reduced hospitalization	None	18	Yes	6
43	Female	Muzafarabad	19.5	No	No	Yes	No	Yes	Yes	No	Yes	Renal	Severe	Yes	Metronidazole	Yes	0	Unrelated	Oral capsule	Successful	Yes	4.66	5.12	Negative	Negative	7627	1.94	3.09	Persistent infection	Improved quality of life	Other	15	No	2
46	Female	Muzafarabad	37.1	No	Yes	Yes	Yes	No	Yes	Yes	No	Renal	Moderate	Yes	Metronidazole	No	3	Unrelated	Oral capsule	Partially successful	Yes	2.88	7.72	Negative	Negative	9446	9.94	2.45	Persistent infection	Reduced hospitalization	None	18	No	24
53	Male	Muzafarabad	31.3	No	No	Yes	Yes	No	No	No	Yes	Neurological	Severe	Yes	None	Yes	2	Related	Enema	Unsuccessful	No	5.28	4.06	Negative	Negative	16657	9.13	3.72	Resolution of infection	Fewer antibiotic uses	None	20	Yes	22
46	Female	Muzafarabad	39	Yes	Yes	Yes	No	Yes	Yes	Yes	Yes	Cardiovascular	Mild	Yes	Vancomycin	No	3	Related	Enema	Unsuccessful	Yes	3.14	7.53	Negative	Positive	5865	14.85	3.75	Persistent infection	Improved quality of life	Mild GI symptoms	3	No	22
66	Female	Muzafarabad	31.3	Yes	Yes	No	Yes	Yes	Yes	No	No	Neurological	Mild	Yes	Metronidazole	Yes	3	Anonymous	Enema	Partially successful	No	4.19	4.78	Positive	Negative	10077	9.15	2.6	Recurrence	Reduced hospitalization	None	30	No	24
71	Male	Muzafarabad	27.3	Yes	No	Yes	Yes	Yes	No	Yes	Yes	Respiratory	Moderate	No	None	No	2	Unrelated	Nasogastric tube	Successful	Yes	4.32	5.42	Negative	Negative	17724	4.68	4.34	Resolution of infection	Fewer antibiotic uses	Other	4	No	5
35	Male	Muzafarabad	26.8	Yes	No	No	Yes	Yes	No	No	Yes	Renal	Severe	Yes	Fidaxomicin	No	2	Related	Enema	Partially successful	Yes	3.13	5.35	Positive	Positive	17391	10.9	3.38	Resolution of infection	Fewer antibiotic uses	Mild GI symptoms	9	Yes	16
68	Male	Muzafarabad	18.3	Yes	Yes	Yes	No	No	No	Yes	No	Renal	Mild	Yes	Vancomycin	Yes	1	Related	Oral capsule	Unsuccessful	Yes	2.48	5.77	Negative	Negative	10516	3.15	4.23	Persistent infection	Reduced hospitalization	Severe infection	3	Yes	19
87	Male	Muzafarabad	36	Yes	No	Yes	No	Yes	No	No	No	Neurological	Mild	No	Fidaxomicin	No	3	Anonymous	Nasogastric tube	Unsuccessful	Yes	3.67	7.35	Positive	Negative	14955	3.24	3.92	Resolution of infection	Fewer antibiotic uses	Other	29	Yes	11
82	Male	Muzafarabad	36.8	Yes	Yes	Yes	No	Yes	No	No	No	Renal	Mild	No	None	Yes	2	Related	Nasogastric tube	Partially successful	No	3.85	5.62	Positive	Negative	8307	14.64	2.73	Persistent infection	Fewer antibiotic uses	Other	20	Yes	16
54	Male	Muzafarabad	28.6	No	Yes	No	Yes	No	No	Yes	Yes	Neurological	Mild	Yes	Metronidazole	Yes	0	Related	Colonoscopy	Unsuccessful	No	5.08	5.63	Positive	Negative	10712	10.6	3.86	Recurrence	Fewer antibiotic uses	None	28	Yes	8
55	Female	Muzafarabad	37.1	No	No	Yes	Yes	No	Yes	No	Yes	Respiratory	Mild	No	Fidaxomicin	No	2	Unrelated	Enema	Unsuccessful	No	5.68	5.62	Negative	Positive	14832	7.71	4.25	Persistent infection	Improved quality of life	Severe infection	14	No	11
28	Male	Muzafarabad	38.1	Yes	No	No	No	Yes	No	Yes	Yes	None	Moderate	Yes	Fidaxomicin	No	0	Related	Colonoscopy	Unsuccessful	No	5.73	4.28	Negative	Negative	5124	13.35	3.53	Persistent infection	Reduced hospitalization	Other	2	Yes	3
81	Female	Muzafarabad	39.5	Yes	Yes	No	No	Yes	No	Yes	No	Neurological	Mild	Yes	None	No	0	Unrelated	Enema	Partially successful	No	5.65	4.68	Negative	Positive	13323	3.84	2.64	Recurrence	Reduced hospitalization	None	6	Yes	8
82	Male	Muzafarabad	22.1	No	Yes	Yes	Yes	Yes	No	No	No	Cardiovascular	Mild	Yes	None	No	2	Unrelated	Nasogastric tube	Unsuccessful	Yes	3.26	5.52	Negative	Positive	17107	2.34	2.21	Resolution of Infection	Reduced hospitalization	None	26	Yes	7
65	Male	Muzafarabad	36.9	Yes	Yes	Yes	No	Yes	Yes	No	No	Respiratory	Mild	No	Fidaxomicin	No	0	Unrelated	Nasogastric tube	Successful	Yes	4.76	6.64	Negative	Negative	5980	4.08	2.28	Recurrence	Fewer antibiotic uses	Severe infection	21	No	16
46	Male	Muzafarabad	21.1	Yes	No	Yes	No	Yes	Yes	Yes	Yes	Renal	Severe	Yes	Fidaxomicin	Yes	0	Anonymous	Enema	Successful	No	4.34	4.04	Negative	Negative	14955	6.02	2.63	Recurrence	Fewer antibiotic uses	Severe infection	4	No	6
73	Female	Muzafarabad	23	No	Yes	No	No	No	Yes	Yes	Yes	Neurological	Moderate	Yes	Vancomycin	Yes	0	Unrelated	Colonoscopy	Partially successful	No	2.42	4.78	Negative	Positive	7944	9.52	3.97	Resolution of infection	Fewer antibiotic uses	Other	6	No	20
22	Female	Muzafarabad	25	No	Yes	No	No	Yes	Yes	Yes	No	Respiratory	Mild	Yes	None	No	2	Unrelated	Nasogastric tube	Partially successful	Yes	3.11	4.19	Negative	Negative	11418	12.37	3.25	Recurrence	Reduced hospitalization	None	21	No	5
53	Male	Muzafarabad	30.7	No	No	No	No	No	Yes	No	Yes	Cardiovascular	Moderate	Yes	Fidaxomicin	No	0	Unrelated	Nasogastric tube	Unsuccessful	No	5.98	7.44	Negative	Negative	6333	3.1	2.6	Resolution of infection	Fewer antibiotic uses	Severe infection	29	Yes	22
27	Female	Muzafarabad	30.8	Yes	Yes	Yes	Yes	No	No	No	Yes	Cardiovascular	Severe	Yes	Fidaxomicin	No	0	Unrelated	Nasogastric tube	Unsuccessful	No	4.68	4.61	Positive	Negative	6714	4.14	3.9	Resolution of infection	Improved quality of life	Severe infection	11	No	18
56	Female	Muzafarabad	27.5	No	No	Yes	No	No	No	Yes	No	None	Moderate	Yes	Metronidazole	Yes	2	Related	Enema	Successful	Yes	3.22	6.6	Negative	Positive	12992	13.85	3.81	Resolution of infection	Reduced hospitalization	Mild GI symptoms	16	No	18
60	Female	Muzafarabad	25.1	Yes	Yes	Yes	No	No	Yes	Yes	No	Cardiovascular	Severe	Yes	Vancomycin	Yes	2	Anonymous	Nasogastric tube	Successful	Yes	5.93	4.69	Positive	Negative	11162	13.94	2.31	Persistent infection	Fewer antibiotic uses	Severe infection	2	Yes	20
33	Female	Muzafarabad	18.3	Yes	Yes	Yes	Yes	No	Yes	No	No	Respiratory	Mild	No	None	Yes	0	Anonymous	Nasogastric tube	Successful	No	3.02	5.9	Negative	Positive	10707	6.77	3.16	Resolution of infection	Fewer antibiotic uses	Other	16	No	7
77	Male	Muzafarabad	30	No	No	No	Yes	No	No	Yes	Yes	None	Severe	Yes	Fidaxomicin	Yes	1	Anonymous	Colonoscopy	Unsuccessful	No	2.47	7.17	Positive	Negative	12500	8.69	3.41	Resolution of infection	Fewer antibiotic uses	Mild GI symptoms	27	Yes	4
22	Female	Muzafarabad	27.8	Yes	No	No	Yes	No	Yes	No	No	Respiratory	Mild	Yes	None	Yes	0	Unrelated	Oral capsule	Partially successful	No	4.72	7.16	Negative	Negative	12904	4.53	2.1	Resolution of infection	Improved quality of life	None	11	Yes	6
80	Female	Muzafarabad	19.5	No	Yes	Yes	No	Yes	Yes	Yes	Yes	Cardiovascular	Mild	No	Fidaxomicin	No	3	Unrelated	Enema	Partially successful	No	2.99	6.43	Positive	Negative	5196	0.98	3.49	Recurrence	Improved quality of life	Other	14	No	6
50	Female	Muzafarabad	32.8	Yes	Yes	No	No	No	Yes	No	No	Neurological	Moderate	No	Vancomycin	Yes	1	Unrelated	Oral capsule	Successful	No	2.98	6.22	Positive	Positive	12631	12.22	4.35	Resolution of infection	Fewer antibiotic uses	Other	22	No	15
47	Male	Muzafarabad	20.8	Yes	Yes	Yes	No	Yes	Yes	No	No	Neurological	Moderate	Yes	Metronidazole	No	2	Anonymous	Nasogastric tube	Unsuccessful	Yes	2.45	7.98	Positive	Positive	16587	9.79	2.72	Recurrence	Reduced hospitalization	Other	17	Yes	11
61	Male	Muzafarabad	21.5	Yes	No	Yes	Yes	No	No	No	No	None	Moderate	No	Fidaxomicin	Yes	0	Anonymous	Colonoscopy	Successful	No	3.05	7.68	Negative	Positive	14204	0.85	4.38	Recurrence	Fewer antibiotic uses	Other	4	No	6
56	Female	Muzafarabad	36.4	Yes	Yes	No	No	Yes	No	No	No	Renal	Severe	No	Vancomycin	No	0	Unrelated	Colonoscopy	Successful	Yes	2.05	4.88	Negative	Positive	11788	7.46	3.34	Persistent infection	Fewer antibiotic uses	None	23	No	18
32	Male	Muzafarabad	27.7	Yes	No	No	Yes	No	Yes	No	Yes	Neurological	Mild	Yes	Vancomycin	Yes	0	Anonymous	Nasogastric tube	Unsuccessful	Yes	5.71	5.82	Positive	Negative	12157	11.01	3.25	Persistent infection	Fewer antibiotic uses	Other	3	Yes	18
80	Female	Muzafarabad	19.8	No	Yes	Yes	Yes	No	No	No	Yes	Neurological	Mild	No	Metronidazole	Yes	1	Unrelated	Nasogastric tube	Partially successful	Yes	5.77	6.68	Positive	Negative	13120	12.5	4.03	Resolution of infection	Improved quality of life	Mild GI symptoms	10	No	21
44	Male	Muzafarabad	34.2	No	Yes	Yes	No	Yes	No	No	No	Cardiovascular	Severe	No	Fidaxomicin	No	2	Unrelated	Colonoscopy	Successful	Yes	5.2	7.94	Negative	Negative	9305	11.7	2.59	Resolution of infection	Improved quality of life	Severe infection	21	No	19
61	Female	Muzafarabad	36.7	Yes	Yes	Yes	No	Yes	Yes	No	Yes	Cardiovascular	Moderate	No	Metronidazole	No	1	Unrelated	Nasogastric tube	Successful	Yes	4.61	4.63	Positive	Positive	10195	14.03	4.38	Recurrence	Improved quality of life	None	3	No	6
42	Female	Muzafarabad	29	No	No	Yes	Yes	No	Yes	Yes	Yes	Respiratory	Severe	Yes	Fidaxomicin	No	0	Unrelated	Enema	Unsuccessful	Yes	2.67	7.18	Negative	Positive	15531	0.53	4.43	Persistent infection	Reduced Hospitalization	None	16	No	24
22	Female	Muzafarabad	27.5	No	No	No	No	Yes	No	Yes	No	Neurological	Moderate	No	None	Yes	0	Related	Nasogastric tube	Partially successful	No	3.74	4.29	Positive	Negative	10658	12.83	3.59	Recurrence	Improved quality of life	Mild GI symptoms	26	Yes	13
23	Female	Muzafarabad	19.3	No	Yes	Yes	Yes	No	No	Yes	Yes	Cardiovascular	Moderate	No	Fidaxomicin	Yes	2	Unrelated	Oral capsule	Successful	No	3.49	5.36	Negative	Negative	11238	5.53	2.79	Recurrence	Fewer antibiotic uses	None	24	No	13
69	Female	Muzafarabad	32	No	No	No	Yes	No	No	No	Yes	Neurological	Severe	No	Fidaxomicin	Yes	0	Related	Oral capsule	Successful	Yes	3.56	6.03	Positive	Positive	12169	3.87	2.12	Persistent infection	Reduced Hospitalization	None	8	Yes	23
77	Male	Muzafarabad	39.7	Yes	No	Yes	No	Yes	No	No	Yes	Cardiovascular	Moderate	Yes	Fidaxomicin	Yes	2	Anonymous	Oral capsule	Partially successful	Yes	3.85	7.37	Negative	Negative	17294	1.33	4	Resolution of infection	Fewer antibiotic uses	Other	7	No	2
35	Male	Muzafarabad	29.8	No	Yes	No	Yes	Yes	Yes	Yes	Yes	Respiratory	Mild	Yes	Metronidazole	Yes	3	Related	Oral capsule	Unsuccessful	No	3.29	5.72	Positive	Positive	5582	10.41	2.41	Resolution of infection	Fewer antibiotic uses	Other	19	Yes	11
58	Female	Muzafarabad	36.2	Yes	No	No	No	Yes	No	No	Yes	None	Moderate	No	Fidaxomicin	Yes	1	Related	Oral capsule	Unsuccessful	No	3.75	5.19	Positive	Negative	14272	6.15	4	Recurrence	Reduced hospitalization	Severe infection	2	No	3
39	Male	Muzafarabad	23.6	No	No	Yes	Yes	No	No	No	Yes	None	Severe	Yes	Fidaxomicin	No	3	Anonymous	Nasogastric tube	Successful	Yes	3.08	6.16	Negative	Negative	10713	12.81	3.13	Recurrence	Improved quality of life	Mild GI symptoms	18	Yes	24
79	Male	Muzafarabad	21.1	No	No	No	Yes	Yes	No	Yes	Yes	Cardiovascular	Severe	No	Vancomycin	No	0	Anonymous	Enema	Partially successful	Yes	5.08	5.02	Negative	Positive	6738	9.24	3.38	Recurrence	Improved quality of life	Other	19	Yes	23
67	Female	Muzafarabad	30.3	Yes	Yes	No	Yes	Yes	No	Yes	Yes	Renal	Moderate	Yes	Vancomycin	Yes	0	Related	Colonoscopy	Partially successful	Yes	4.18	7.79	Negative	Positive	4401	10.31	3.82	Persistent infection	Improved quality of life	Other	26	No	6
18	Male	Muzafarabad	30.7	Yes	No	No	Yes	No	No	No	Yes	Cardiovascular	Severe	Yes	None	Yes	0	Anonymous	Enema	Unsuccessful	Yes	2.35	7.89	Negative	Positive	6223	12.17	2.98	Resolution of infection	Improved quality of life	None	18	Yes	4
82	Male	Muzafarabad	36.2	Yes	Yes	Yes	Yes	Yes	No	No	Yes	None	Moderate	Yes	Vancomycin	Yes	0	Anonymous	Colonoscopy	Partially successful	No	5.15	6.43	Positive	Positive	5516	7.4	2.59	Persistent infection	Fewer antibiotic uses	Other	23	No	5
25	Female	Muzafarabad	33.3	No	No	Yes	No	Yes	Yes	No	Yes	Renal	Severe	Yes	Fidaxomicin	No	0	Unrelated	Enema	Successful	Yes	4.48	7.49	Positive	Positive	15421	9.81	3.75	Recurrence	Improved quality of life	None	19	Yes	21
33	Female	Muzafarabad	34.6	No	Yes	Yes	Yes	No	No	No	Yes	Respiratory	Mild	Yes	Fidaxomicin	No	3	Unrelated	Enema	Partially successful	Yes	2.34	6.54	Negative	Negative	16026	3.18	3.06	Recurrence	Reduced hospitalization	Other	8	No	15
32	Female	Muzafarabad	28.8	No	No	Yes	No	Yes	No	No	Yes	Renal	Mild	Yes	Fidaxomicin	No	0	Anonymous	Enema	Successful	No	4.88	5.3	Positive	Positive	7631	8.12	2.63	Persistent infection	Improved quality of life	None	14	No	22
74	Female	Muzafarabad	38.7	No	Yes	Yes	Yes	No	Yes	Yes	No	Neurological	Mild	Yes	Fidaxomicin	No	0	Anonymous	Colonoscopy	Successful	No	4.58	6.57	Negative	Negative	10623	10.87	2.38	Persistent infection	Fewer antibiotic uses	Mild GI symptoms	16	Yes	19
29	Male	Muzafarabad	34.2	Yes	No	No	Yes	No	No	No	Yes	None	Moderate	No	Metronidazole	No	2	Related	Enema	Unsuccessful	Yes	3.42	5.91	Negative	Negative	12284	13.98	2.8	Resolution of infection	Fewer antibiotic uses	Other	8	No	16
39	Male	Muzafarabad	39.5	Yes	No	No	No	Yes	No	No	No	Neurological	Moderate	Yes	Fidaxomicin	No	3	Anonymous	Oral capsule	Successful	Yes	5.18	5.76	Negative	Negative	17181	0.79	3.56	Recurrence	Improved quality of life	Mild GI symptoms	8	No	11
89	Female	Muzafarabad	23.4	Yes	Yes	Yes	No	No	No	Yes	Yes	None	Mild	Yes	Metronidazole	No	2	Anonymous	Enema	Partially successful	No	5.74	6.39	Negative	Positive	5981	8.32	3.49	Resolution of infection	Improved quality of life	Mild GI symptoms	8	Yes	13
25	Male	Muzafarabad	23.6	Yes	Yes	Yes	No	No	Yes	No	Yes	Respiratory	Mild	Yes	Metronidazole	No	0	Unrelated	Enema	Partially successful	Yes	2.79	5.5	Negative	Negative	9611	15	3.79	Resolution of infection	Fewer antibiotic uses	None	18	No	21
38	Male	Muzafarabad	32.9	No	Yes	Yes	Yes	No	No	No	No	Neurological	Mild	Yes	Vancomycin	Yes	1	Related	Oral capsule	Partially successful	No	4.72	4.92	Negative	Negative	4094	1.4	3.58	Recurrence	Improved quality of life	None	22	Yes	3
20	Male	Muzafarabad	32.9	No	No	Yes	No	Yes	No	Yes	Yes	Neurological	Mild	No	Vancomycin	Yes	2	Related	Enema	Successful	Yes	4.63	5.79	Negative	Positive	13880	7.99	2.53	Resolution of infection	Improved quality of life	None	6	No	19
29	Male	Muzafarabad	20	Yes	No	No	Yes	Yes	Yes	No	Yes	Cardiovascular	Mild	No	Vancomycin	Yes	0	Anonymous	Enema	Successful	Yes	4.19	4.65	Negative	Negative	14555	0.82	2.93	Persistent infection	Fewer antibiotic uses	None	26	Yes	11
65	Male	Muzafarabad	25.2	Yes	Yes	Yes	Yes	No	Yes	No	Yes	Cardiovascular	Severe	No	None	No	2	Unrelated	Nasogastric tube	Successful	Yes	4.35	4.63	Positive	Negative	14226	1.14	3.74	Persistent infection	Fewer antibiotic uses	None	8	No	17
70	Female	Muzafarabad	34.2	Yes	No	Yes	No	No	No	No	Yes	Neurological	Moderate	Yes	Metronidazole	No	0	Related	Colonoscopy	Partially successful	Yes	2.74	4.12	Positive	Positive	12763	10.48	3.34	Resolution of infection	Fewer antibiotic uses	Other	4	No	23
41	Female	Muzafarabad	25.5	No	Yes	Yes	Yes	Yes	No	No	No	Cardiovascular	Moderate	No	Fidaxomicin	Yes	0	Unrelated	Nasogastric tube	Successful	Yes	5.04	4.57	Negative	Positive	9840	6.59	2.06	Recurrence	Fewer antibiotic uses	None	3	Yes	12
78	Male	Muzafarabad	35	No	No	Yes	Yes	Yes	No	Yes	Yes	Respiratory	Mild	Yes	Metronidazole	No	1	Related	Colonoscopy	Unsuccessful	Yes	3.29	4.37	Negative	Positive	17792	4.39	3.06	Resolution of infection	Improved quality of life	Mild GI symptoms	23	No	3
58	Male	Muzafarabad	36.6	Yes	Yes	Yes	No	Yes	Yes	Yes	Yes	Cardiovascular	Moderate	No	Vancomycin	No	1	Related	Colonoscopy	Unsuccessful	Yes	3.65	7.84	Negative	Negative	9016	3.28	4.46	Persistent infection	Reduced hospitalization	None	9	Yes	13
75	Female	Muzafarabad	26.9	No	No	No	No	Yes	Yes	No	Yes	Renal	Severe	No	Metronidazole	No	0	Anonymous	Nasogastric tube	Partially successful	No	4.67	7.15	Positive	Negative	12853	3.37	3.56	Resolution of infection	Reduced hospitalization	Severe infection	7	No	13
81	Female	Muzafarabad	27.7	Yes	Yes	Yes	No	No	Yes	No	Yes	Renal	Moderate	No	Metronidazole	Yes	2	Anonymous	Nasogastric tube	Unsuccessful	Yes	5.77	4.95	Positive	Negative	7320	5.56	3.72	Resolution of infection	Improved quality of life	Other	16	Yes	9
47	Female	Muzafarabad	38.9	Yes	Yes	No	No	Yes	No	No	Yes	Neurological	Moderate	No	Fidaxomicin	No	2	Related	Colonoscopy	Successful	Yes	2.78	5.08	Negative	Positive	9622	14.11	4.22	Recurrence	Fewer antibiotic uses	Other	15	No	9
73	Male	Muzafarabad	31.5	No	Yes	Yes	Yes	Yes	Yes	No	No	Cardiovascular	Mild	No	Fidaxomicin	No	0	Related	Nasogastric tube	Unsuccessful	Yes	5.15	6.01	Positive	Positive	17184	12.05	2.51	Recurrence	Reduced hospitalization	Other	25	Yes	7
87	Male	Muzafarabad	30.2	No	No	Yes	Yes	Yes	No	No	Yes	Renal	Moderate	No	Fidaxomicin	Yes	2	Related	Colonoscopy	Successful	No	5.58	4.15	Negative	Negative	14274	14.73	3.8	Recurrence	Reduced hospitalization	None	23	No	1
20	Female	Muzafarabad	30.6	No	No	No	Yes	No	No	No	No	Respiratory	Severe	Yes	Vancomycin	Yes	2	Related	Nasogastric tube	Successful	Yes	3.19	7.63	Positive	Positive	14000	2.17	2.62	Persistent infection	Improved quality of life	Severe infection	9	No	24
20	Female	Muzafarabad	31.6	No	No	Yes	Yes	No	Yes	No	No	Renal	Mild	Yes	Metronidazole	Yes	0	Unrelated	Enema	Partially successful	No	3.51	4.43	Positive	Negative	17141	12.33	4.42	Recurrence	Improved quality of life	Severe infection	6	No	3
72	Male	Muzafarabad	21.3	Yes	Yes	Yes	No	Yes	No	Yes	Yes	None	Mild	Yes	Metronidazole	Yes	1	Related	Enema	Unsuccessful	Yes	2.74	6.31	Negative	Negative	11610	3.53	4.21	Resolution of infection	Fewer antibiotic uses	Mild GI symptoms	11	No	7
63	Female	Muzafarabad	33.6	No	Yes	No	No	No	No	Yes	Yes	None	Severe	No	Vancomycin	Yes	1	Anonymous	Nasogastric tube	Partially successful	No	3.49	4.28	Positive	Negative	4546	8.14	4.21	Recurrence	Improved quality of life	Other	20	Yes	22
40	Male	Muzafarabad	36.5	No	No	Yes	Yes	Yes	Yes	No	Yes	Renal	Severe	No	Fidaxomicin	No	1	Related	Nasogastric tube	Partially successful	Yes	3.05	4.86	Negative	Positive	6158	2.07	2.35	Recurrence	Fewer antibiotic uses	Other	28	Yes	22
82	Female	Muzafarabad	22.2	Yes	Yes	No	Yes	No	Yes	Yes	Yes	None	Moderate	Yes	Fidaxomicin	Yes	3	Unrelated	Oral capsule	Unsuccessful	Yes	3.63	7.14	Positive	Negative	14757	2.37	4.3	Recurrence	Fewer antibiotic uses	Mild GI symptoms	6	Yes	12
26	Female	Muzafarabad	21.8	Yes	No	No	No	Yes	No	Yes	No	Neurological	Severe	No	None	No	2	Anonymous	Nasogastric tube	Successful	No	5.32	5.68	Positive	Negative	14621	14.73	2.21	Resolution of infection	Reduced hospitalization	Other	23	Yes	19
86	Male	Muzafarabad	39.8	No	Yes	No	Yes	No	No	Yes	Yes	Respiratory	Moderate	No	Fidaxomicin	Yes	3	Unrelated	Colonoscopy	Partially successful	Yes	3.88	6.15	Positive	Positive	14159	7.91	4.3	Recurrence	Reduced hospitalization	Mild GI symptoms	18	No	4
72	Male	Muzafarabad	20.4	No	Yes	Yes	Yes	Yes	No	No	Yes	Renal	Moderate	No	None	Yes	0	Related	Oral capsule	Successful	No	4.39	4.73	Positive	Negative	9125	2.25	3.73	Persistent infection	Improved quality of life	Severe infection	13	No	23
77	Male	Muzafarabad	34.3	No	Yes	No	No	No	No	No	No	Renal	Moderate	No	Vancomycin	No	0	Unrelated	Nasogastric tube	Partially successful	Yes	5.09	6.26	Positive	Positive	10117	3.87	4.43	Persistent infection	Improved quality of life	Other	21	No	9
26	Female	Muzafarabad	31.9	Yes	No	No	Yes	Yes	Yes	Yes	Yes	Renal	Severe	Yes	Metronidazole	Yes	2	Unrelated	Oral capsule	Partially successful	No	5.89	4.18	Negative	Negative	12515	14.43	4.07	Resolution of infection	Reduced hospitalization	None	9	No	22
52	Female	Muzafarabad	22.5	No	No	Yes	Yes	No	Yes	No	Yes	Respiratory	Severe	Yes	None	No	2	Anonymous	Enema	Successful	No	5.62	6.16	Positive	Negative	10930	8.76	4.06	Recurrence	Improved quality of life	Severe infection	22	No	1
77	Female	Muzafarabad	22.7	No	Yes	Yes	No	Yes	No	No	Yes	None	Mild	Yes	Fidaxomicin	No	2	Unrelated	Enema	Partially successful	Yes	3.58	5.92	Positive	Positive	11412	2.46	2.01	Recurrence	Fewer antibiotic uses	Other	28	No	12
33	Female	Muzafarabad	24	Yes	Yes	Yes	No	Yes	No	Yes	Yes	Renal	Severe	Yes	None	Yes	0	Unrelated	Oral capsule	Partially successful	Yes	2.18	6.95	Negative	Positive	10722	7.04	3.84	Recurrence	Improved quality of life	Severe infection	18	No	9
41	Male	Muzafarabad	20.8	No	Yes	Yes	Yes	No	No	Yes	Yes	None	Mild	Yes	Vancomycin	Yes	3	Unrelated	Nasogastric tube	Partially successful	Yes	2.09	5.77	Negative	Negative	16409	5.09	3.96	Recurrence	Reduced hospitalization	Other	12	No	18
45	Male	Muzafarabad	24.8	Yes	No	Yes	No	Yes	No	No	Yes	Neurological	Severe	No	Vancomycin	Yes	1	Unrelated	Nasogastric tube	Unsuccessful	Yes	2.3	4.68	Negative	Positive	11821	2.65	2.99	Persistent infection	Improved quality of life	Other	22	Yes	23
61	Male	Muzafarabad	32.8	No	No	Yes	No	Yes	No	Yes	No	None	Severe	No	None	Yes	1	Related	Colonoscopy	Unsuccessful	No	3.54	7.81	Positive	Positive	9095	5.71	3.77	Persistent infection	Fewer antibiotic uses	Severe infection	28	No	14
59	Male	Muzafarabad	26.4	Yes	Yes	No	No	No	Yes	No	Yes	Respiratory	Moderate	No	Vancomycin	No	0	Anonymous	Oral capsule	Unsuccessful	Yes	4.67	6.23	Negative	Positive	13328	10.13	2.08	Recurrence	Improved quality of life	None	30	Yes	17
66	Male	Muzafarabad	23	Yes	Yes	No	No	No	No	Yes	Yes	Respiratory	Mild	No	Fidaxomicin	No	3	Unrelated	Nasogastric tube	Unsuccessful	Yes	3.13	7.88	Negative	Positive	16137	11.69	2.74	Recurrence	Fewer antibiotic uses	Other	16	No	17
77	Male	Muzafarabad	32.9	No	No	No	No	No	Yes	Yes	No	Cardiovascular	Mild	No	Fidaxomicin	No	3	Related	Colonoscopy	Successful	Yes	2.49	4.22	Positive	Positive	16364	9.01	2.43	Resolution of infection	Improved quality of life	Severe infection	10	Yes	1
54	Male	Muzafarabad	29.2	Yes	Yes	Yes	No	No	Yes	No	Yes	Cardiovascular	Severe	Yes	None	No	0	Unrelated	Colonoscopy	Partially successful	No	4.87	4.92	Negative	Negative	12669	14.08	3.53	Resolution of infection	Improved quality of life	Other	29	Yes	23
25	Female	Muzafarabad	23.4	No	No	Yes	No	No	No	Yes	Yes	Neurological	Mild	No	Metronidazole	Yes	1	Related	Nasogastric tube	Successful	Yes	3.61	6.92	Negative	Positive	7270	1.05	3.98	Resolution of infection	Reduced hospitalization	Severe infection	30	Yes	22
31	Male	Muzafarabad	39.6	Yes	Yes	No	Yes	Yes	Yes	No	No	Neurological	Severe	No	Vancomycin	No	2	Anonymous	Enema	Unsuccessful	No	3.24	6.23	Negative	Positive	7887	3.96	2.77	Persistent infection	Fewer antibiotic uses	Mild GI symptoms	14	Yes	6
29	Male	Muzafarabad	38.5	No	No	No	No	No	No	Yes	Yes	None	Mild	Yes	Metronidazole	Yes	1	Unrelated	Colonoscopy	Successful	No	2.43	4.27	Negative	Negative	8984	8.62	4.12	Resolution of infection	Fewer antibiotic uses	Other	17	No	8
85	Female	Muzafarabad	27.8	No	No	Yes	No	No	Yes	Yes	No	Cardiovascular	Moderate	Yes	None	Yes	1	Anonymous	Oral capsule	Successful	Yes	3.82	5.18	Positive	Negative	7473	2.85	4.42	Persistent infection	Reduced hospitalization	Severe infection	6	No	10
40	Female	Muzafarabad	25.6	No	Yes	No	Yes	No	No	No	Yes	None	Moderate	Yes	Vancomycin	No	0	Related	Colonoscopy	Partially successful	No	4.19	6.37	Negative	Positive	17119	5.9	2.3	Recurrence	Fewer antibiotic uses	Mild GI symptoms	18	No	3
52	Male	Muzafarabad	38.7	No	Yes	No	No	No	No	No	No	Renal	Mild	No	Fidaxomicin	No	3	Unrelated	Colonoscopy	Successful	Yes	5.41	7.79	Negative	Negative	10462	6.03	3.83	Resolution of infection	Fewer antibiotic uses	None	27	Yes	6
77	Female	Muzafarabad	33.4	Yes	Yes	Yes	Yes	Yes	No	Yes	Yes	Cardiovascular	Moderate	Yes	Vancomycin	Yes	0	Related	Enema	Unsuccessful	No	2.46	4.03	Positive	Negative	16891	2.51	3.78	Resolution of infection	Reduced hospitalization	Severe infection	12	Yes	3
68	Male	Muzafarabad	21.4	Yes	Yes	No	Yes	No	Yes	No	No	Respiratory	Moderate	No	Metronidazole	No	2	Unrelated	Enema	Successful	Yes	4.74	5.19	Positive	Positive	10877	5.06	2.01	Persistent infection	Reduced hospitalization	Severe infection	30	No	4
88	Female	Muzafarabad	20.1	No	No	No	No	No	No	No	No	Cardiovascular	Moderate	Yes	Fidaxomicin	No	0	Anonymous	Enema	Partially successful	No	4.66	6.2	Negative	Negative	15613	12.05	2.68	Persistent infection	Reduced hospitalization	Mild GI symptoms	29	Yes	24
44	Male	Muzafarabad	33.9	No	No	Yes	Yes	No	No	No	No	Renal	Severe	No	None	No	0	Unrelated	Nasogastric tube	Partially successful	No	4.51	6.82	Positive	Negative	13951	2.41	4.26	Recurrence	Reduced hospitalization	Mild GI symptoms	22	Yes	20
34	Male	Muzafarabad	34.8	Yes	Yes	No	Yes	No	No	No	No	Neurological	Mild	No	Vancomycin	No	0	Unrelated	Nasogastric tube	Unsuccessful	No	2.47	5.37	Positive	Positive	5844	9.11	4.4	Resolution of infection	Improved quality of life	None	9	No	10
85	Female	Muzafarabad	31.4	No	No	No	No	Yes	Yes	No	Yes	Respiratory	Mild	Yes	Metronidazole	Yes	2	Anonymous	Colonoscopy	Successful	Yes	2.89	6	Negative	Positive	8706	9.2	4.44	Recurrence	Reduced hospitalization	Other	21	Yes	19
51	Female	Muzafarabad	31.7	Yes	Yes	Yes	No	No	No	No	Yes	Respiratory	Severe	No	None	Yes	1	Anonymous	Oral capsule	Successful	No	3.25	4.48	Positive	Negative	10322	1.34	2.83	Persistent infection	Improved quality of life	Other	14	No	3
83	Male	Muzafarabad	21.6	Yes	No	No	No	Yes	No	No	No	None	Moderate	No	None	Yes	1	Anonymous	Enema	Successful	Yes	2.95	7.77	Negative	Negative	17985	3.95	3.79	Recurrence	Reduced hospitalization	Other	19	No	23
87	Female	Muzafarabad	18.7	No	Yes	No	No	No	Yes	Yes	Yes	None	Severe	Yes	Vancomycin	No	0	Unrelated	Oral capsule	Partially successful	No	3.11	4.74	Positive	Negative	11725	3.64	3.47	Resolution of infection	Improved quality of life	None	28	Yes	2
74	Female	Muzafarabad	40	Yes	Yes	No	Yes	Yes	No	No	Yes	Cardiovascular	Moderate	No	Metronidazole	No	1	Related	Enema	Successful	Yes	4.6	4.99	Positive	Positive	9342	1.99	4.08	Persistent infection	Reduced hospitalization	Mild GI symptoms	29	No	8
76	Male	Muzafarabad	35.6	No	Yes	No	No	No	No	No	Yes	Respiratory	Mild	No	Vancomycin	No	3	Unrelated	Enema	Partially successful	No	2.93	4.71	Positive	Negative	4595	7.39	4.3	Recurrence	Reduced hospitalization	None	6	Yes	3
71	Female	Muzafarabad	36.9	Yes	No	No	No	Yes	No	No	Yes	Renal	Severe	Yes	Metronidazole	Yes	1	Anonymous	Oral capsule	Partially successful	Yes	4.73	6.11	Positive	Positive	9508	1.89	3.77	Persistent infection	Fewer antibiotic uses	Severe infection	20	Yes	8
37	Female	Muzafarabad	25.1	No	Yes	Yes	Yes	No	Yes	No	Yes	Renal	Mild	No	None	No	1	Anonymous	Oral capsule	Unsuccessful	Yes	2.97	5.25	Negative	Positive	8393	8.66	2.48	Recurrence	Improved quality of life	Mild GI symptoms	21	No	23
64	Female	Muzafarabad	31.7	Yes	No	Yes	Yes	No	No	Yes	No	Cardiovascular	Severe	No	Fidaxomicin	No	3	Related	Colonoscopy	Partially successful	No	5.05	6.07	Negative	Positive	6808	9.26	2.05	Persistent infection	Fewer antibiotic uses	Other	29	No	23
35	Male	Muzafarabad	22.6	Yes	Yes	No	No	No	Yes	Yes	Yes	Neurological	Severe	No	Metronidazole	No	3	Unrelated	Colonoscopy	Unsuccessful	Yes	3.3	5.96	Negative	Negative	16203	6.26	3.34	Resolution of infection	Reduced hospitalization	Mild GI symptoms	17	Yes	5
84	Female	Muzafarabad	29.2	No	No	No	Yes	Yes	Yes	No	No	Renal	Severe	Yes	None	No	3	Anonymous	Enema	Unsuccessful	Yes	2.92	7.03	Negative	Negative	6498	5.53	2.93	Persistent infection	Reduced hospitalization	Other	19	Yes	19
76	Female	Muzafarabad	39	Yes	Yes	Yes	No	Yes	No	Yes	No	Cardiovascular	Severe	No	Fidaxomicin	Yes	0	Anonymous	Oral capsule	Successful	No	5.3	4.48	Positive	Positive	16439	3.83	2.1	Resolution of infection	Improved quality of life	Severe infection	21	Yes	3
61	Male	Muzafarabad	35	Yes	No	Yes	No	No	No	Yes	Yes	Neurological	Severe	No	Fidaxomicin	No	2	Related	Enema	Successful	No	4.57	4.1	Positive	Positive	10517	7.29	3.03	Recurrence	Improved quality of life	Other	2	No	23
43	Male	Muzafarabad	22	Yes	Yes	No	Yes	No	No	No	No	Cardiovascular	Moderate	Yes	None	Yes	1	Anonymous	Nasogastric tube	Partially successful	No	4.61	6.82	Positive	Positive	9627	2.75	3.37	Resolution of infection	Improved quality of life	Severe infection	20	Yes	19
57	Female	Muzafarabad	31.6	Yes	Yes	No	Yes	No	Yes	No	Yes	Renal	Moderate	No	Metronidazole	Yes	3	Unrelated	Enema	Unsuccessful	No	4.85	5.88	Negative	Positive	11270	11.6	2.53	Recurrence	Fewer antibiotic uses	Severe infection	11	No	4
45	Male	Muzafarabad	38.9	Yes	Yes	Yes	No	No	No	Yes	No	Neurological	Severe	Yes	None	Yes	0	Anonymous	Oral capsule	Unsuccessful	No	3.11	5.92	Negative	Negative	5510	7.65	3.73	Persistent infection	Reduced hospitalization	None	12	Yes	3
87	Female	Muzafarabad	21.6	No	Yes	No	No	Yes	No	No	No	Neurological	Severe	No	None	Yes	2	Unrelated	Enema	Unsuccessful	No	3.29	4.42	Positive	Negative	11674	14.53	2.68	Recurrence	Reduced hospitalization	Mild GI symptoms	15	No	24
33	Female	Muzafarabad	33.8	Yes	No	Yes	Yes	No	No	No	Yes	Renal	Moderate	No	Vancomycin	Yes	1	Unrelated	Enema	Unsuccessful	Yes	4.9	7.28	Negative	Negative	5838	2.71	2.68	Persistent infection	Reduced hospitalization	Other	4	No	23
61	Male	Muzafarabad	19.3	Yes	No	No	No	No	No	Yes	No	Cardiovascular	Mild	No	Metronidazole	No	0	Unrelated	Nasogastric tube	Partially successful	No	3	5.53	Negative	Negative	5581	6.99	3.25	Persistent infection	Improved quality of life	Severe infection	5	Yes	7
41	Male	Muzafarabad	26.4	Yes	Yes	Yes	No	No	Yes	No	No	Respiratory	Moderate	No	None	Yes	2	Related	Colonoscopy	Unsuccessful	Yes	3.27	4.48	Positive	Positive	17143	13.36	3.25	Persistent Infection	Improved quality of life	Severe infection	2	No	6
89	Female	Muzafarabad	22.1	Yes	No	No	Yes	No	No	Yes	No	Neurological	Mild	Yes	Vancomycin	Yes	1	Anonymous	Colonoscopy	Partially successful	Yes	3.16	4.84	Positive	Negative	14649	13.94	2.52	Recurrence	Reduced Hospitalization	Other	2	No	12
78	Female	Muzafarabad	29.1	Yes	No	Yes	Yes	No	Yes	Yes	No	Cardiovascular	Mild	Yes	Vancomycin	No	0	Related	Nasogastric tube	Partially Successful	No	4.8	6.94	Negative	Positive	8068	11	3.57	Persistent infection	Reduced hospitalization	Other	29	No	23
35	Female	Muzafarabad	35.7	No	Yes	No	Yes	No	No	No	Yes	Neurological	Mild	Yes	Vancomycin	No	0	Unrelated	Nasogastric tube	Successful	No	2.62	6.51	Negative	Positive	14604	12.24	3.04	Persistent infection	Reduced hospitalization	Severe infection	2	No	2
31	Male	Muzafarabad	18.1	No	Yes	Yes	Yes	Yes	Yes	No	No	None	Mild	Yes	Fidaxomicin	No	0	Unrelated	Nasogastric tube	Partially successful	Yes	3.95	6.11	Negative	Positive	10286	6.93	4.18	Resolution of infection	Fewer antibiotic uses	Other	30	No	24
69	Female	Muzafarabad	25.6	Yes	No	Yes	Yes	No	No	Yes	No	None	Moderate	No	Metronidazole	No	0	Anonymous	Colonoscopy	Unsuccessful	Yes	2.15	4.55	Positive	Positive	15979	10.99	2.87	Resolution of infection	Fewer antibiotic uses	Other	5	No	24
32	Male	Muzafarabad	27.6	Yes	No	Yes	Yes	No	Yes	No	Yes	Cardiovascular	Moderate	No	None	No	0	Anonymous	Nasogastric tube	Unsuccessful	No	4	4.65	Positive	Negative	9848	10.65	2.9	Resolution of infection	Reduced hospitalization	Other	5	Yes	11
63	Female	Muzafarabad	37.8	No	Yes	Yes	Yes	No	Yes	No	No	Renal	Mild	No	None	Yes	2	Unrelated	Nasogastric tube	Partially successful	Yes	2.03	7.82	Negative	Positive	14303	2.63	3.86	Persistent infection	Reduced hospitalization	Mild GI symptoms	30	No	1
50	Female	Muzafarabad	33	No	No	No	No	No	No	No	No	Cardiovascular	Moderate	Yes	Fidaxomicin	No	3	Anonymous	Colonoscopy	Successful	No	2.5	6.64	Positive	Positive	15780	5.24	2.1	Persistent infection	Fewer antibiotic uses	None	3	Yes	13
84	Female	Muzafarabad	27.2	Yes	No	No	No	Yes	No	Yes	Yes	Respiratory	Moderate	No	Metronidazole	Yes	1	Anonymous	Enema	Unsuccessful	No	3.72	7.67	Negative	Positive	9927	14.76	3.49	Resolution of infection	Reduced hospitalization	Other	27	No	20
73	Female	Muzafarabad	20	No	No	Yes	No	Yes	Yes	Yes	No	None	Moderate	Yes	Vancomycin	Yes	2	Anonymous	Oral capsule	Partially successful	Yes	5.1	4.12	Positive	Negative	9436	10.06	3.8	Recurrence	Improved quality of life	Severe infection	6	No	22
86	Female	Muzafarabad	31.5	No	No	Yes	No	Yes	No	No	No	Renal	Severe	Yes	Metronidazole	No	2	Unrelated	Colonoscopy	Successful	Yes	2.89	7.27	Positive	Positive	6926	3.5	2.49	Resolution of infection	Reduced hospitalization	None	18	No	11
78	Female	Muzafarabad	24.6	Yes	No	No	No	Yes	No	No	No	Renal	Moderate	Yes	Vancomycin	Yes	1	Anonymous	Nasogastric tube	Unsuccessful	Yes	3.49	6.55	Negative	Positive	11786	3.12	4.1	Resolution of infection	Fewer antibiotic uses	Severe infection	5	No	22
60	Female	Muzafarabad	33.9	Yes	No	No	Yes	No	No	Yes	Yes	Neurological	Moderate	Yes	Fidaxomicin	Yes	0	Anonymous	Colonoscopy	Successful	Yes	5.51	4.03	Negative	Negative	13733	5.49	3.53	Resolution of infection	Reduced hospitalization	Mild GI symptoms	19	No	9
70	Male	Muzafarabad	19.8	Yes	No	Yes	Yes	No	Yes	No	Yes	Renal	Mild	No	Vancomycin	Yes	3	Related	Colonoscopy	Unsuccessful	No	2.2	4.71	Positive	Negative	6533	6.23	4	Resolution of infection	Fewer antibiotic uses	Severe infection	10	No	7
42	Male	Muzafarabad	20.9	Yes	Yes	Yes	No	No	No	No	No	Respiratory	Severe	No	Metronidazole	No	1	Related	Oral capsule	Successful	No	5.82	7.68	Positive	Positive	11447	0.71	3.34	Resolution of infection	Fewer antibiotic uses	None	13	No	11
54	Male	Muzafarabad	27.4	Yes	Yes	Yes	Yes	Yes	Yes	Yes	Yes	Renal	Moderate	No	Metronidazole	No	0	Related	Colonoscopy	Successful	Yes	4.7	6.59	Negative	Positive	6330	12.2	3.97	Resolution of infection	Fewer antibiotic uses	Other	24	Yes	13
35	Female	Muzafarabad	24.2	Yes	Yes	No	Yes	No	No	Yes	Yes	None	Severe	Yes	Vancomycin	Yes	0	Unrelated	Enema	Partially successful	No	5.25	6.03	Negative	Positive	17360	14.51	4.31	Resolution of infection	Fewer antibiotic uses	Mild GI symptoms	30	No	6
42	Male	Muzafarabad	19.2	No	Yes	Yes	Yes	Yes	Yes	Yes	No	Neurological	Mild	No	Vancomycin	No	0	Related	Colonoscopy	Unsuccessful	No	5.67	4.03	Positive	Negative	10022	13.21	2.55	Persistent infection	Fewer antibiotic uses	None	25	Yes	10
25	Female	Muzafarabad	32.9	Yes	No	No	No	No	No	No	No	Respiratory	Moderate	Yes	Vancomycin	No	0	Related	Colonoscopy	Unsuccessful	Yes	5.57	6.99	Negative	Positive	12838	14.87	3.59	Recurrence	Reduced hospitalization	Other	12	Yes	20
57	Male	Muzafarabad	30.9	Yes	Yes	Yes	Yes	Yes	No	Yes	Yes	Renal	Moderate	Yes	Metronidazole	Yes	2	Anonymous	Nasogastric tube	Unsuccessful	Yes	4.45	6.15	Negative	Negative	10583	4.26	3.35	Recurrence	Improved quality of life	Mild GI symptoms	29	No	21
29	Female	Muzafarabad	37.7	Yes	No	No	No	Yes	No	No	No	Respiratory	Mild	No	Fidaxomicin	No	0	Related	Oral capsule	Unsuccessful	No	4.94	5.25	Positive	Positive	7179	5.98	3.71	Persistent infection	Reduced hospitalization	Other	5	Yes	13
85	Female	Muzafarabad	38.6	Yes	Yes	No	No	No	Yes	Yes	Yes	Neurological	Severe	Yes	Metronidazole	No	0	Anonymous	Oral capsule	Unsuccessful	No	5.11	4.76	Positive	Negative	17280	7.09	3.86	Recurrence	Improved quality of life	Severe infection	6	No	11
66	Male	Muzafarabad	37.5	No	No	Yes	No	Yes	Yes	No	No	Respiratory	Moderate	Yes	Fidaxomicin	Yes	0	Unrelated	Oral capsule	Unsuccessful	No	2.19	7.78	Positive	Negative	10157	14.7	4.45	Persistent infection	Reduced hospitalization	Mild GI symptoms	18	Yes	8
32	Female	Muzafarabad	27.5	No	No	Yes	Yes	No	No	No	Yes	Neurological	Severe	Yes	Fidaxomicin	Yes	0	Related	Colonoscopy	Unsuccessful	Yes	5.13	6.42	Positive	Negative	5732	0.96	2.59	Persistent infection	Fewer antibiotic uses	Mild GI symptoms	17	No	23
29	Male	Muzafarabad	31.9	No	Yes	Yes	No	No	Yes	No	Yes	Neurological	Mild	No	Metronidazole	Yes	0	Related	Nasogastric tube	Successful	Yes	2.71	7.06	Positive	Positive	4936	4.77	4.14	Resolution of infection	Fewer antibiotic uses	Severe infection	21	No	21
80	Male	Muzafarabad	25.4	Yes	Yes	No	No	Yes	Yes	No	No	Neurological	Severe	Yes	None	No	2	Related	Oral capsule	Successful	No	4.22	6.35	Positive	Positive	16729	3.33	4.33	Persistent infection	Reduced hospitalization	Severe infection	15	No	11
88	Male	Muzafarabad	37.4	Yes	No	No	Yes	No	Yes	No	No	Neurological	Mild	No	Metronidazole	Yes	3	Related	Oral capsule	Unsuccessful	Yes	3.69	5.11	Positive	Positive	9710	2.98	3.76	Recurrence	Fewer antibiotic uses	None	14	Yes	23
85	Female	Muzafarabad	20.9	No	No	No	No	No	No	Yes	Yes	Respiratory	Mild	Yes	Vancomycin	Yes	2	Anonymous	Nasogastric tube	Successful	No	5.19	7.16	Negative	Negative	17929	3.49	3.44	Resolution of infection	Improved quality of life	Mild GI symptoms	23	No	7
29	Male	Muzafarabad	22.4	No	Yes	No	No	No	No	No	No	None	Mild	Yes	Metronidazole	No	0	Anonymous	Enema	Successful	No	2.11	5.02	Negative	Positive	6527	5.4	2.33	Persistent infection	Improved quality of life	Mild GI symptoms	23	Yes	13
40	Female	Muzafarabad	31.1	Yes	No	No	No	No	Yes	No	Yes	Neurological	Moderate	Yes	Metronidazole	Yes	1	Unrelated	Oral capsule	Partially successful	No	5.95	6.48	Negative	Negative	11858	0.82	3.22	Resolution of infection	Improved quality of life	Other	19	No	4
67	Male	Muzafarabad	36.1	No	Yes	Yes	No	Yes	No	No	Yes	None	Moderate	No	Metronidazole	No	3	Unrelated	Enema	Unsuccessful	No	2.82	6.41	Positive	Negative	4943	1.14	4.2	Resolution of infection	Reduced hospitalization	Other	18	No	2
88	Female	Muzafarabad	39.5	Yes	No	No	Yes	No	Yes	No	No	Renal	Mild	Yes	None	Yes	0	Unrelated	Colonoscopy	Successful	No	2.24	6.36	Negative	Negative	16233	1.84	3.99	Resolution of infection	Improved quality of life	None	23	No	21
38	Female	Muzafarabad	25.4	Yes	Yes	Yes	Yes	No	No	Yes	Yes	None	Moderate	Yes	Vancomycin	No	3	Related	Oral capsule	Successful	Yes	5.32	5.37	Positive	Positive	7755	6.3	3.77	Recurrence	Improved quality of life	Mild GI symptoms	11	Yes	9
40	Female	Muzafarabad	38.4	Yes	Yes	Yes	No	No	No	No	Yes	None	Severe	No	None	Yes	0	Anonymous	Enema	Successful	No	5.42	6.37	Negative	Positive	9327	6.94	3.91	Persistent infection	Fewer antibiotic uses	None	13	Yes	2
40	Female	Muzafarabad	20.7	Yes	Yes	Yes	No	No	Yes	No	Yes	Respiratory	Severe	Yes	Vancomycin	No	2	Anonymous	Enema	Partially successful	Yes	2.06	7.26	Positive	Positive	11268	3.5	4.24	Persistent infection	Fewer antibiotic uses	Mild GI symptoms	5	No	1
42	Female	Muzafarabad	39.5	Yes	Yes	Yes	Yes	No	No	No	Yes	Neurological	Mild	Yes	Metronidazole	Yes	3	Unrelated	Enema	Successful	No	4.38	4.35	Positive	Positive	14482	5.75	2.82	Persistent infection	Fewer antibiotic uses	Other	29	No	6
48	Female	Muzafarabad	36.3	No	Yes	Yes	Yes	Yes	No	No	No	Neurological	Mild	No	Metronidazole	Yes	0	Anonymous	Oral capsule	Unsuccessful	Yes	2.89	4.89	Positive	Positive	15232	3.97	3.96	Persistent infection	Reduced hospitalization	Mild GI symptoms	15	Yes	22
83	Male	Muzafarabad	22.2	No	No	Yes	Yes	No	No	No	No	Renal	Moderate	No	Fidaxomicin	Yes	2	Unrelated	Nasogastric tube	Partially successful	Yes	3.09	6.08	Positive	Negative	8100	10.54	3.18	Persistent infection	Fewer antibiotic uses	Mild GI symptoms	8	No	8
19	Male	Muzafarabad	37.5	No	No	Yes	Yes	No	Yes	No	No	Respiratory	Moderate	Yes	None	No	0	Related	Colonoscopy	Successful	No	3.68	5	Negative	Positive	11130	14.58	4.19	Persistent infection	Improved quality of life	Other	3	Yes	1
77	Male	Muzafarabad	34.8	Yes	Yes	No	Yes	Yes	No	No	No	Neurological	Mild	Yes	Fidaxomicin	No	0	Unrelated	Enema	Partially successful	No	3.35	7.89	Negative	Positive	14595	10.51	3.07	Recurrence	Reduced hospitalization	Mild GI symptoms	13	Yes	22
82	Male	Muzafarabad	26.6	Yes	No	No	No	Yes	Yes	No	Yes	None	Severe	Yes	None	No	0	Related	Oral capsule	Unsuccessful	Yes	5.99	7.34	Negative	Negative	8393	1.79	2.09	Persistent infection	Improved quality of life	None	15	Yes	24
33	Male	Muzafarabad	28.4	No	Yes	Yes	No	No	No	Yes	Yes	None	Mild	No	Vancomycin	Yes	1	Related	Oral capsule	Unsuccessful	Yes	4.46	4.99	Negative	Positive	7855	6.08	2.68	Resolution of infection	Improved quality of life	None	3	No	21
25	Male	Muzafarabad	23.1	No	No	Yes	Yes	No	Yes	No	No	Neurological	Severe	Yes	Vancomycin	No	0	Related	Enema	Partially successful	No	2.47	7.71	Positive	Negative	10581	4.8	3.1	Persistent infection	Improved quality of life	None	3	Yes	21
23	Female	Muzafarabad	37.6	No	Yes	Yes	No	Yes	Yes	Yes	No	None	Severe	Yes	Metronidazole	No	0	Anonymous	Colonoscopy	Unsuccessful	Yes	4.32	6.75	Negative	Positive	7520	8.61	3.91	Recurrence	Reduced hospitalization	Other	15	No	13
32	Female	Muzafarabad	34.9	Yes	No	Yes	No	Yes	No	No	No	Neurological	Severe	Yes	Vancomycin	Yes	1	Anonymous	Nasogastric tube	Successful	No	3.43	4.1	Negative	Positive	16567	1.99	3.71	Recurrence	Reduced hospitalization	Severe infection	26	No	4
45	Female	Muzafarabad	28.8	Yes	Yes	No	No	Yes	No	No	Yes	Cardiovascular	Mild	No	Fidaxomicin	No	2	Related	Nasogastric tube	Partially successful	No	5.79	7.91	Negative	Positive	7082	8.38	3.62	Recurrence	Fewer antibiotic uses	Severe infection	10	No	11
23	Female	Muzafarabad	36.9	No	Yes	No	Yes	Yes	Yes	No	No	Cardiovascular	Severe	Yes	None	No	1	Unrelated	Colonoscopy	Partially successful	Yes	3.33	5.8	Negative	Positive	10136	13.05	3.19	Persistent infection	Fewer antibiotic uses	Severe infection	10	Yes	16
75	Female	Muzafarabad	23	Yes	Yes	No	No	Yes	No	Yes	No	Renal	Severe	Yes	None	Yes	1	Unrelated	Nasogastric tube	Unsuccessful	Yes	3.74	5.1	Negative	Positive	8025	10.23	4.2	Persistent infection	Improved quality of life	None	9	No	18
49	Male	Muzafarabad	32.2	Yes	Yes	No	No	No	Yes	No	Yes	Respiratory	Mild	Yes	Vancomycin	No	0	Unrelated	Oral capsule	Successful	No	3.44	6.18	Negative	Positive	6778	1.97	4.12	Persistent infection	Reduced hospitalization	Other	14	No	20
24	Female	Muzafarabad	20.9	Yes	Yes	No	Yes	No	No	No	Yes	Renal	Mild	No	None	Yes	3	Related	Oral capsule	Partially successful	No	2.01	5.51	Negative	Positive	12779	3.48	2.93	Persistent infection	Reduced hospitalization	None	12	Yes	2
61	Male	Muzafarabad	22.7	No	No	No	No	No	No	Yes	Yes	Respiratory	Severe	No	Metronidazole	Yes	3	Related	Oral capsule	Unsuccessful	Yes	5.01	4.79	Positive	Negative	12839	9.39	4.47	Recurrence	Fewer antibiotic uses	Other	7	No	20
66	Female	Muzafarabad	20.2	Yes	Yes	Yes	No	No	Yes	Yes	No	Respiratory	Severe	No	Fidaxomicin	No	3	Unrelated	Nasogastric tube	Partially successful	Yes	5.1	5.46	Negative	Negative	11396	9.78	3.93	Resolution of infection	Fewer antibiotic uses	Severe infection	30	Yes	24
59	Male	Muzafarabad	38.6	No	No	No	No	Yes	No	No	Yes	Cardiovascular	Severe	Yes	Fidaxomicin	Yes	0	Unrelated	Colonoscopy	Unsuccessful	No	5.03	6.29	Negative	Positive	5138	10.72	2.97	Persistent infection	Fewer antibiotic uses	None	15	No	21
42	Male	Muzafarabad	35.1	Yes	Yes	Yes	No	Yes	No	Yes	Yes	Renal	Severe	Yes	Vancomycin	Yes	1	Anonymous	Nasogastric tube	Unsuccessful	No	4.28	5.98	Positive	Negative	16304	5.27	2.06	Persistent infection	Improved quality of life	Severe infection	24	Yes	11
59	Female	Muzafarabad	27.2	Yes	Yes	Yes	Yes	Yes	Yes	No	No	None	Moderate	No	Metronidazole	No	0	Related	Colonoscopy	Successful	No	2.39	4.25	Positive	Positive	14120	0.65	2.78	Resolution of infection	Fewer antibiotic uses	Mild GI symptoms	30	No	12
90	Female	Muzafarabad	28	No	Yes	No	No	Yes	Yes	No	No	None	Severe	Yes	Fidaxomicin	Yes	0	Unrelated	Nasogastric tube	Unsuccessful	Yes	2.6	4.27	Negative	Negative	11094	2.43	2.03	Persistent infection	Fewer antibiotic uses	Severe infection	25	Yes	16
57	Female	Muzafarabad	23.8	No	No	No	No	No	Yes	No	Yes	Cardiovascular	Severe	Yes	Fidaxomicin	Yes	0	Anonymous	Oral capsule	Unsuccessful	Yes	5.33	5.74	Positive	Positive	6869	4.45	2.02	Persistent infection	Fewer antibiotic uses	Mild GI symptoms	10	No	23
90	Female	Muzafarabad	28.7	Yes	No	Yes	Yes	No	Yes	No	Yes	Renal	Moderate	Yes	Fidaxomicin	No	0	Related	Nasogastric tube	Successful	No	2.37	6.22	Positive	Positive	4139	0.61	3.87	Resolution of infection	Reduced hospitalization	Severe infection	17	No	16
25	Male	Muzafarabad	37.3	No	No	Yes	Yes	Yes	No	Yes	Yes	Neurological	Severe	Yes	Metronidazole	No	0	Unrelated	Colonoscopy	Unsuccessful	No	4.99	4.66	Positive	Negative	14251	9.77	2.08	Recurrence	Fewer antibiotic uses	Severe infection	12	No	12
27	Male	Muzafarabad	34.9	No	Yes	No	No	Yes	Yes	No	Yes	Respiratory	Moderate	No	None	Yes	1	Related	Nasogastric tube	Partially successful	No	2.92	6.51	Positive	Negative	14938	0.62	3.53	Resolution of infection	Fewer antibiotic uses	None	2	No	22
88	Male	Muzafarabad	19	Yes	Yes	No	No	No	No	No	Yes	Respiratory	Moderate	Yes	Fidaxomicin	Yes	0	Anonymous	Enema	Partially successful	No	3.09	5.18	Negative	Negative	11247	9.88	3.04	Persistent infection	Reduced hospitalization	Other	10	Yes	10
22	Female	Muzafarabad	35.5	Yes	Yes	No	Yes	Yes	No	No	Yes	Cardiovascular	Mild	Yes	Vancomycin	Yes	0	Anonymous	Oral capsule	Partially successful	Yes	4.96	7.75	Negative	Negative	5652	12.19	2.58	Resolution of infection	Improved quality of life	None	25	No	15
70	Female	Muzafarabad	30.5	Yes	Yes	Yes	Yes	Yes	Yes	Yes	Yes	Neurological	Severe	Yes	Vancomycin	No	0	Anonymous	Oral capsule	Unsuccessful	No	5.66	5.19	Positive	Positive	14131	12.29	3.55	Resolution of infection	Improved quality of life	Other	13	No	6
52	Female	Muzafarabad	30.7	No	No	No	No	Yes	Yes	Yes	No	Renal	Severe	No	Metronidazole	No	1	Related	Colonoscopy	Unsuccessful	Yes	2.89	4.84	Negative	Negative	5667	13.91	3.18	Persistent infection	Improved quality of life	Mild GI symptoms	22	No	4
83	Female	Muzafarabad	32.2	Yes	Yes	Yes	No	No	Yes	No	No	Neurological	Severe	No	None	No	2	Related	Enema	Unsuccessful	Yes	4.11	6.56	Negative	Negative	7152	4.16	3.53	Resolution of infection	Reduced hospitalization	Severe infection	12	No	1
72	Male	Muzafarabad	34.3	Yes	No	Yes	No	No	No	No	Yes	None	Moderate	Yes	Fidaxomicin	Yes	0	Related	Enema	Unsuccessful	No	3.78	4.48	Positive	Negative	8825	5.34	3.79	Recurrence	Improved quality of life	Severe infection	6	Yes	10
71	Female	Muzafarabad	36.3	Yes	No	No	No	Yes	No	No	No	Renal	Moderate	No	None	Yes	2	Unrelated	Enema	Unsuccessful	No	2.22	4.48	Positive	Positive	6414	1.65	3.16	Persistent infection	Fewer antibiotic uses	None	11	No	15
84	Male	Muzafarabad	26.5	Yes	Yes	Yes	No	Yes	No	Yes	Yes	Cardiovascular	Severe	No	Metronidazole	No	0	Unrelated	Enema	Partially successful	No	5.23	6.24	Positive	Positive	16452	1.98	3.42	Recurrence	Fewer antibiotic uses	None	11	Yes	21
78	Male	Muzafarabad	18.9	Yes	No	No	Yes	No	No	Yes	No	Cardiovascular	Severe	No	Metronidazole	No	2	Related	Enema	Successful	No	2.34	5.5	Negative	Positive	17065	8.21	2.5	Persistent infection	Fewer antibiotic uses	Severe infection	16	No	17
63	Female	Muzafarabad	19.4	No	No	No	No	Yes	Yes	Yes	No	Neurological	Mild	No	Fidaxomicin	No	3	Unrelated	Colonoscopy	Partially successful	No	3.47	7.18	Positive	Negative	10979	10.63	3.7	Resolution of infection	Improved quality of life	None	18	No	13
72	Male	Muzafarabad	31.4	No	Yes	No	Yes	Yes	Yes	No	No	Renal	Mild	No	Fidaxomicin	Yes	1	Unrelated	Enema	Successful	No	4.62	4.57	Positive	Negative	7458	1.89	3.37	Resolution of infection	Improved quality of life	Other	11	Yes	13
69	Female	Muzafarabad	32.3	Yes	No	Yes	No	No	Yes	Yes	No	Respiratory	Severe	No	Fidaxomicin	No	3	Unrelated	Enema	Unsuccessful	Yes	2.58	6.03	Negative	Positive	5312	14.52	4.13	Persistent infection	Improved quality of life	Other	28	Yes	14
76	Male	Muzafarabad	35.2	Yes	Yes	Yes	No	No	Yes	Yes	Yes	Renal	Moderate	No	Metronidazole	No	0	Unrelated	Nasogastric tube	Partially successful	No	3.49	4.26	Positive	Positive	11860	0.6	3.4	Recurrence	Reduced hospitalization	Severe infection	11	Yes	14
75	Female	Muzafarabad	18.7	No	No	No	Yes	Yes	Yes	Yes	No	Renal	Severe	Yes	None	Yes	0	Related	Nasogastric tube	Partially successful	No	3.99	6.78	Positive	Negative	10189	7.68	3.34	Persistent infection	Improved quality of life	Other	21	Yes	23
26	Male	Muzafarabad	38.5	No	Yes	No	Yes	No	Yes	Yes	Yes	Respiratory	Moderate	Yes	Fidaxomicin	Yes	2	Related	Oral capsule	Unsuccessful	Yes	5.62	5.29	Negative	Negative	14221	12.76	2.77	Recurrence	Improved quality of life	None	3	Yes	17
71	Male	Muzafarabad	30.8	No	No	Yes	Yes	Yes	Yes	Yes	Yes	None	Mild	No	Fidaxomicin	Yes	2	Unrelated	Nasogastric tube	Successful	Yes	3.87	5.95	Positive	Negative	15813	5.53	4.16	Persistent infection	Reduced hospitalization	None	5	No	8
50	Male	Muzafarabad	29.2	No	No	No	Yes	No	Yes	Yes	Yes	Cardiovascular	Severe	No	Vancomycin	No	0	Unrelated	Colonoscopy	Successful	Yes	4.6	5.68	Positive	Negative	9438	10.03	3.66	Resolution of infection	Reduced hospitalization	Mild GI symptoms	19	Yes	23
88	Male	Muzafarabad	22.8	Yes	No	No	Yes	Yes	Yes	Yes	Yes	Cardiovascular	Mild	No	None	Yes	3	Related	Nasogastric tube	Unsuccessful	Yes	2.86	7.81	Negative	Positive	6052	7.39	4.43	Persistent infection	Fewer antibiotic uses	Other	30	No	12
65	Female	Muzafarabad	36.1	Yes	Yes	Yes	No	No	No	No	No	Renal	Severe	No	Fidaxomicin	Yes	0	Related	Colonoscopy	Unsuccessful	Yes	4.08	5.73	Positive	Positive	4053	9.84	4.14	Persistent infection	Reduced hospitalization	None	30	No	7
36	Male	Muzafarabad	35.4	Yes	No	Yes	No	No	Yes	No	No	Cardiovascular	Moderate	Yes	Vancomycin	No	0	Anonymous	Colonoscopy	Successful	Yes	3.63	6.86	Positive	Negative	17517	9.91	4.17	Persistent infection	Fewer antibiotic uses	Severe infection	22	Yes	24
27	Female	Muzafarabad	25.9	No	Yes	No	No	No	No	No	No	None	Mild	Yes	Fidaxomicin	No	0	Unrelated	Nasogastric tube	Successful	No	2.98	4.64	Negative	Negative	12887	6.13	4.31	Recurrence	Improved quality of life	None	24	Yes	4
20	Female	Muzafarabad	39.7	Yes	Yes	Yes	No	Yes	No	Yes	No	Neurological	Mild	No	Vancomycin	Yes	1	Unrelated	Nasogastric tube	Successful	Yes	3.08	6.49	Positive	Negative	12930	0.98	3.93	Resolution of infection	Improved quality of life	Other	12	No	16
75	Female	Muzafarabad	22.8	No	Yes	Yes	Yes	Yes	Yes	Yes	No	Renal	Severe	No	Metronidazole	Yes	0	Anonymous	Oral capsule	Partially successful	Yes	2.69	5.87	Positive	Negative	7840	8.56	2.38	Resolution of infection	Reduced hospitalization	Mild GI symptoms	13	Yes	22
65	Female	Muzafarabad	37.5	No	Yes	Yes	Yes	No	Yes	No	No	Cardiovascular	Moderate	Yes	Metronidazole	Yes	3	Unrelated	Colonoscopy	Successful	Yes	5.67	6.63	Positive	Positive	11832	2.27	2.76	Resolution of infection	Improved quality of life	Mild GI symptoms	16	No	8
72	Male	Muzafarabad	19.8	Yes	Yes	No	Yes	No	No	Yes	No	Respiratory	Severe	Yes	None	No	0	Anonymous	Nasogastric tube	Unsuccessful	Yes	2.73	5.24	Positive	Positive	5426	5.06	2	Recurrence	Reduced hospitalization	Severe infection	8	No	14
61	Female	Muzafarabad	24.6	Yes	Yes	No	Yes	No	No	No	Yes	Cardiovascular	Moderate	Yes	Fidaxomicin	No	0	Anonymous	Colonoscopy	Unsuccessful	No	4.98	6.18	Negative	Negative	12574	6.72	2.26	Recurrence	Fewer antibiotic uses	None	23	Yes	17
46	Female	Muzafarabad	25.5	Yes	No	No	No	No	Yes	Yes	Yes	Neurological	Moderate	No	Metronidazole	No	2	Anonymous	Nasogastric tube	Unsuccessful	Yes	5.5	7.01	Negative	Negative	14106	6.72	3.14	Persistent infection	Reduced hospitalization	Other	26	No	15
61	Male	Muzafarabad	18.9	No	No	No	No	Yes	Yes	No	No	Neurological	Severe	Yes	Vancomycin	Yes	3	Related	Nasogastric tube	Successful	No	4.02	4.89	Negative	Positive	12574	6.68	4.38	Persistent infection	Fewer antibiotic uses	Mild GI symptoms	15	No	4
87	Male	Muzafarabad	30.8	Yes	Yes	Yes	No	Yes	Yes	Yes	No	None	Mild	Yes	Metronidazole	Yes	0	Unrelated	Oral capsule	Successful	No	4.74	5.86	Positive	Negative	5776	10.46	2.12	Persistent infection	Improved quality of life	Mild GI symptoms	11	No	17
62	Female	Muzafarabad	21	No	Yes	No	No	No	No	No	No	Neurological	Severe	Yes	Metronidazole	No	2	Anonymous	Nasogastric tube	Successful	No	4.9	6.32	Positive	Negative	9090	3.48	4.01	Resolution of ifection	Fewer antibiotic uses	None	21	Yes	21
32	Male	Muzafarabad	22.2	Yes	Yes	No	Yes	Yes	No	No	Yes	Neurological	Severe	Yes	Fidaxomicin	Yes	3	Unrelated	Colonoscopy	Successful	No	3.96	5.29	Positive	Positive	16352	5.18	3.78	Recurrence	Reduced hospitalization	Other	26	No	9
62	Male	Muzafarabad	18.9	Yes	Yes	No	No	Yes	No	Yes	Yes	Renal	Moderate	No	None	Yes	1	Related	Nasogastric tube	Successful	Yes	5.13	5.75	Positive	Positive	4833	14.98	3.97	Persistent infection	Fewer antibiotic uses	Severe infection	15	Yes	8
29	Female	Muzafarabad	33.8	Yes	Yes	No	Yes	Yes	Yes	No	No	Respiratory	Mild	Yes	Fidaxomicin	Yes	0	Anonymous	Nasogastric tube	Unsuccessful	Yes	4.46	7.25	Positive	Negative	8662	12.28	2.16	Resolution of infection	Fewer antibiotic uses	Severe infection	15	No	22
52	Male	Muzafarabad	28.8	No	No	No	No	No	No	Yes	No	Renal	Mild	No	Vancomycin	Yes	0	Related	Enema	Successful	Yes	4.45	7.09	Negative	Negative	17514	11.75	2.72	Recurrence	Fewer antibiotic uses	Other	8	No	12
29	Female	Muzafarabad	39.1	Yes	Yes	Yes	Yes	Yes	No	Yes	No	None	Mild	Yes	None	Yes	0	Related	Colonoscopy	Unsuccessful	No	4.43	6.13	Positive	Positive	11290	13.38	2.8	Resolution of infection	Fewer antibiotic uses	Other	11	No	16
85	Female	Muzafarabad	32.5	Yes	No	Yes	Yes	Yes	Yes	Yes	No	Neurological	Moderate	Yes	Vancomycin	No	0	Anonymous	Enema	Unsuccessful	No	2.91	4.44	Positive	Positive	16973	11.07	2.73	Persistent infection	Fewer antibiotic uses	Other	13	Yes	15
83	Male	Muzafarabad	27.5	Yes	Yes	No	Yes	No	No	Yes	No	Cardiovascular	Severe	Yes	Metronidazole	Yes	0	Related	Oral capsule	Partially successful	Yes	3.15	6.43	Positive	Negative	11283	2.05	2.87	Persistent infection	Fewer antibiotic uses	Severe infection	27	No	15
33	Male	Muzafarabad	20	No	Yes	Yes	No	No	No	No	No	Cardiovascular	Mild	Yes	Metronidazole	Yes	0	Anonymous	Oral capsule	Partially successful	Yes	5.5	6.87	Negative	Positive	9528	13.56	3.72	Recurrence	Improved quality of life	Mild GI symptoms	19	Yes	22
81	Male	Muzafarabad	24.2	Yes	Yes	Yes	Yes	Yes	Yes	Yes	No	Renal	Severe	Yes	None	No	0	Anonymous	Oral capsule	Unsuccessful	No	4.89	7.62	Positive	Positive	16310	8.23	4.42	Persistent infection	Reduced hjospitalization	Mild GI symptoms	12	No	1
47	Male	Muzafarabad	24.7	No	Yes	No	No	No	No	Yes	Yes	Renal	Severe	No	Metronidazole	Yes	0	Related	Colonoscopy	Partially successful	No	4.25	5.43	Negative	Negative	10422	8.62	2.8	Persistent infection	Fewer antibiotic Uses	None	26	No	15
32	Female	Muzafarabad	37.9	No	No	Yes	No	No	Yes	Yes	Yes	Renal	Mild	No	Metronidazole	Yes	3	Unrelated	Colonoscopy	Unsuccessful	Yes	2.66	4.76	Negative	Negative	16502	10.75	4.1	Resolution of infection	Improved quality of life	Severe infection	14	No	9
59	Male	Muzafarabad	23.6	No	No	No	Yes	No	Yes	No	No	Neurological	Mild	No	Metronidazole	Yes	1	Unrelated	Colonoscopy	Successful	No	4.43	6.03	Negative	Negative	8105	10.88	2.25	Recurrence	Improved quality of life	Severe infection	7	Yes	5
32	Male	Muzafarabad	36.8	Yes	No	Yes	No	No	Yes	No	Yes	None	Moderate	Yes	Vancomycin	No	3	Anonymous	Enema	Partially successful	Yes	3.4	5.51	Positive	Negative	11323	4.61	2.13	Persistent infection	Improved quality of life	Other	21	No	15
40	Male	Muzafarabad	22.2	No	Yes	Yes	Yes	No	No	Yes	No	Neurological	Severe	Yes	Metronidazole	No	0	Unrelated	Colonoscopy	Successful	Yes	5.83	6.84	Positive	Negative	5403	8.03	3.41	Resolution of infection	Improved quality of life	None	20	Yes	11
87	Male	Muzafarabad	31.8	Yes	Yes	Yes	Yes	No	No	No	No	Cardiovascular	Severe	Yes	Metronidazole	No	1	Anonymous	Oral capsule	Successful	No	5.57	7.8	Negative	Negative	5367	8.93	2.28	Resolution of infection	Improved quality of life	Severe infection	26	Yes	18
76	Male	Muzafarabad	35.5	No	Yes	No	Yes	No	No	No	Yes	Renal	Severe	Yes	Vancomycin	No	0	Unrelated	Enema	Partially successful	No	4.75	4.53	Negative	Negative	7941	6.67	3.84	Resolution of infection	Improved quality of life	None	10	Yes	9
51	Male	Muzafarabad	23.9	Yes	Yes	Yes	Yes	Yes	Yes	No	Yes	Neurological	Moderate	No	None	Yes	0	Related	Colonoscopy	Partially successful	No	5.28	5.19	Negative	Negative	4040	7.33	3.82	Recurrence	Fewer antibiotic uses	Severe infection	13	No	7
